This article has been retracted.

# Novel Decision-Making Techniques in Tripolar Fuzzy Environment with Application: A Case Study of ERP Systems

**DOI:** 10.1155/2022/4488576

**Published:** 2022-01-31

**Authors:** Minhaj Afridi, Abdu H. Gumaei, Hussain AlSalman, Asghar Khan, Sk. Md. Mizanur Rahman

**Affiliations:** ^1^Department of Mathematics, Faculty of Physical and Numerical Sciences, Abdul Wali Khan University, Mardan, Khyber Pakhtunkhwa, Pakistan; ^2^Department of Computer Science, Faculty of Applied Sciences, Taiz University, Taiz 6803, Yemen; ^3^Department of Computer Science, College of Computer and Information Sciences, King Saud University, Riyadh 11543, Saudi Arabia; ^4^Information and Communication Engineering Technology, School of Engineering Technology and Applied Science, Centennial College, Toronto, Canada

## Abstract

The intuitionistic fuzzy set (IFS) and bipolar fuzzy set (BFS) are all effective models to describe ambiguous and incomplete cognitive knowledge with membership, non-membership, negative membership, and hesitancy sections. But in daily life problems, there are some situations where we cannot apply the ordinary models of IFS and BFS, separately. Hence, there is a need to combine both the models of IFS and BFS into a single one. A tripolar fuzzy set (TFS) is a generalization of IFS and BFS. In circumstances where BFS and IFS models cannot be used individually, a tripolar fuzzy model is more dependable and efficient. Further, the IFS and BFS models are reduced to corollaries due to the proposed model of TFS. For this purpose in this article, we first consider some novel operations on tripolar fuzzy information. These operations are formulated on the basis of well-known Dombi T-norm and T-conorm, and the desirable properties are discussed. By applying the Dombi operations, arithmetic and geometric aggregation operators of TFS are proposed, and we introduce the concepts of a TF-Dombi weighted average (TFDWA) operator, a TF-Dombi ordered weighted average (TFDOWA) operator, and a TF-Dombi hybrid weighted (TFDHW) operator and explore their fundamental features including idempotency, boundedness, monotonicity, and others. In the second part, we propose TF-Dombi weighted geometric (TFDWG) operator, TF-Dombi ordered weighted geometric (TFDOWG) operator, and TF-Dombi hybrid geometric (TFDHG) operator. The features and specific cases of the mentioned operators are examined. Enterprise resource planning (ERP) is a management and integration approach that organizations employ to manage and develop many aspects of their operations. The study's primary contribution is to employ TFS to create certain decision-making strategies for the selection of optimal ERP systems. The proposed operators are then used to build several techniques for solving multiattribute decision-making (MADM) issues with TF information. Finally, an example of ERP system selection is investigated to demonstrate that the techniques suggested are trustworthy and realistic.

## 1. Introduction

Decision making (DM) is a method of resolving real-world problems by selecting the ideal choice from a range of viable options. MADM is an area of operations research in which the best answer is found after weighing all of the options against a set of criteria. In real life, there are numerous challenges that are ambiguous and uncertain. To deal with uncertain and ambiguous information. Zadeh developed fuzzy set (FS) theory [1]. The idea of intuitionistic fuzzy set (IFS) developed by Atanassov [2, 3] comprised two degree membership functions, namely, accepting and denying. IFS is a potential generalization of the notion of a FS [1], whose degree component contained only accepting degree. Decision science is a continuously growing ground in the modern technological era. In the decision process, experts select an optimal alternative under some preference values imposed by the experts in a given finite set of alternatives. Decision-making methods have been used in several areas of modern science, for example, Xu [4] developed the use of IFS in arithmetic aggregation operators (AOPs) and initiated many valuable operators. Afterwards, Xu and Yager [5] developed some geometric AOPs and demonstrated the use of these operators in MADM. Since its inception, the IFS has attracted a lot of interest, including dynamic MADM in the IF setting [6, 7], IF aggregation operators [8–13], IF entropy [14–16], IF generalized Dice similarity measures [16], IF TOPSIS [14–16], and IF gray relational analysis [17–19]. Many generalizations of IFS were developed in the literature after the successful stages of IFS. The bipolar fuzzy set (BFS) [20, 21] was developed to measure the uncertain and cognitive information presented in the form of positive polarity and negative polarity in real-world scenarios. The objects in a universe in BFS are characterized by positive polarity and negative polarity, and the BFS has range of membership in [−1,1]. Chen et al. [22] studied an empirical examination of attribute interrelationships that are heterogeneous in a MADM. For MADM, a unique consensus model based on multigranular HFLTSs was established in [23]. In [24], a method was developed and implemented in MADM issues to present a linguistic distribution assessment (LDA) using a hesitant linguistic distribution (HLD). A new strategy for dealing with MCGDM problems with unbalanced HFLTSs was established in [25] taking psychological behaviour of DMs. The notion of a BFS has been employed in many potential areas including bipolar logical reasoning and other set theoretical abstract structures [20], theoretical approach to traditional medicine of China [26], computational psychiatry [27], decision analysis and organizational modeling [28], and quantum computing [29]. Recently, Dombi [30] studied decision methods by developing some arithmetic and geometric AOPs with the help of Dombi operations and BFSs. The topics in fuzzy information aggregation operators are developing rapidly, and many researchers are involved to construct feasible and advanced models to deal with decision processes. In [31], Liu applied Hamăcher AOPs in interval-valued IF numbers (IVIFNs) and constructed MAGDM methods. Wang and Garg [32] defined some Pythagorean fuzzy interaction aggregation operators with the aid of Archimedean t-conorm and t-norm (ATT) to aggregate the numbers. Zhang [33] proposed IVIFNs in Frank AOPs and considered the applications in MAGDM. Zhang and Zhang [34] defined Einstein hybrid AOPs for IFNs and applied it to the MADM method.

A new fuzzy extension has just been developed, dubbed tripolar FS (TFS), which is a generalization of IFS and BFS [35]. In instances where IFS and BFS models are difficult to apply, a TF model can be used. In TFS, we consider a triplet of real numbers, namely, the membership, non-membership, and negative membership degrees, which is used to define an object in a TFS. Similar to BFS, the range of membership of the TFS is also [−1,1]. A TFS model can easily be applied in situations where IFS and BFS models fail.

Wei [8] developed several novel operations known as Dombi T-norm (DTN) and Dombi T-conorm (DTCN), which have a high potential for parameter variation. Han et al. [26] took advantage by performing Dombi operations on IFSs and developing MAGDM problems utilizing the Dombi Bonferroni mean operator and IF information. Wei et al. [21, 36], in a single-valued neutrosophic environment, constructed a MADM problem utilizing Dombi operations. Lu and Busemeyer [27] defined typhoon disaster assessment using Dombi operations in a HF context. In this paper, we presented various AOPs in a TF environment by using an expanded idea of IFS and BFS. The following points describe the novelty of proposed operators:

- The ability of a TFS is to express IFS and BFS information at once in a single notion called tripolar fuzzy environment which makes it exceptional in literature. The qualitative characteristics of IFS and BFS are combined in a single TFS. As a result, the work is presented in a TFS context to deal with tripolarity type of fuzzy information.
- The flexibility parameter involved in Dombi operations has the ability to produce more accurate results in a decision process.
- The proposed model can be applied in situations where the traditional models of IFS and BFS fail.
- Dombi operations' flexible parameter make it simple to investigate the stability of ranking order of alternatives.
- The score function was crucial in creating a ranking order among the choices in DM situations. By integrating the concepts of IFS and BFS score functions, a new concept of score function is constructed in the proposed study.

The rest of the paper is structured as follows.

The essential ideas of the IFS, BFSs, and TFSs, as well as the operational regulations of TFNs, will be addressed in the next section. In Section 3, we established the TF-Dombi weighted average (TFDWA), TF-Dombi ordered weighted average (TFDOWA), TF-Dombi hybrid average (TFDHA), TF-Dombi weighted geometric (TFDWG), TF-Dombi ordered weighted geometric (TFDOWG), and TF-Dombi hybrid geometric (TFDHG) operators. The peculiarities and specific cases of these operators are also explored. In Section 4, we used these operators to come up with some solutions to the TF MADM challenges.  Section 5 examines an illustrated example of ERP system selection. Some remarks are made in Section 6, where we conclude the article.

## 2. Preliminaries

In this section, we review the definitions of IFS, BFS, and TFS extracted from [1–3, 37], and then we construct a novel notion of score and accuracy functions and introduce a new comparison technique for TFS.

**Definition 1 (see [2, 3]).**

An IFS *f* of a non-empty set $\tilde{X}$ is an object of the form

(1) $$\begin{array}{c} \tilde{f}=\langle \mu_{\tilde{f}}^{\cdot },\lambda_{\tilde{f}}^{\cdot }\rangle =\left\{\langle x,\mu_{\tilde{f}}^{\cdot }\left(x\right),\lambda_{\tilde{f}}^{\cdot }\left(x\right)\rangle |x\in \tilde{X}\right\}, \end{array}$$

where $\mu_{\tilde{f}}^{\cdot }:\tilde{X}⟶\left[0,1\right]$ and $\lambda_{\tilde{f}}^{\cdot }:\tilde{X}⟶\left[0,1\right]$ represent the degree of membership and non-membership of an element *x* in FS $\tilde{f}$, respectively, and $0\leq \mu_{\tilde{f}}^{\cdot }\left(x\right)+\lambda_{\tilde{f}}^{\cdot }\left(x\right)\leq 1$ for all $x\in \tilde{X}$.

**Definition 2 (see [37]).**

A BFS *A* of a non-empty set $\tilde{X}$ is an object with a shape

(2) $$\begin{array}{c} \tilde{A}=\langle \mu_{\tilde{A}}^{\cdot },\delta_{\tilde{A}}^{\cdot }\rangle =\left\{\langle x,\mu_{\tilde{A}}^{\cdot }\left(x\right),\delta_{\tilde{A}}^{\cdot }\left(x\right)\rangle |x\in \tilde{X}\right\}, \end{array}$$

where $\mu_{\tilde{A}}^{\cdot }:\tilde{X}⟶\left[0,1\right]$ and $\delta_{\tilde{A}}^{\cdot }:\tilde{X}⟶\left[-1,0\right]$ indicate the degree to which an element *x* satisfies the associated property to BFS $\tilde{A}$, as well as the implicit counter property to BFS $\tilde{A}$ and

(3) $$\begin{array}{c} -1\leq \mu_{\tilde{A}}^{\cdot }\left(x\right)+\delta_{\tilde{A}}^{\cdot }\left(x\right)\leq 1, \end{array}$$

for all $x\in \tilde{X}$.

**Definition 3 (see [35]).**

A TFS $\tilde{A}$ of a non-empty set $\tilde{X}$ is an object

(4) $$\begin{array}{c} \tilde{A}=\langle \mu_{\tilde{A}}^{\cdot },\lambda_{\tilde{A}}^{\cdot },\delta_{\tilde{A}}^{\cdot }\rangle =\left\{\langle x,\mu_{\tilde{A}}^{\cdot }\left(x\right),\lambda_{\tilde{A}}^{\cdot }\left(x\right),\delta_{\tilde{A}}^{\cdot }\left(x\right)\rangle |x\in \tilde{X}\right\}, \end{array}$$

where $\mu_{\tilde{A}}^{\cdot }:\tilde{X}⟶\left[0,1\right]$, $\lambda_{\tilde{A}}^{\cdot }:\tilde{X}⟶\left[0,1\right]$ and $\delta_{\tilde{A}}^{\cdot }:\tilde{X}⟶\left[-1,0\right]$ such that $0\leq \mu_{\tilde{A}}^{\cdot }\left(x\right)+\lambda_{\tilde{A}}^{\cdot }\left(x\right)\leq 1$. The membership degree $\mu_{\tilde{A}}^{\cdot }\left(x\right)$ is the amount to which the element *x* satisfies the condition to the TFS $\tilde{A}$, $\lambda_{\tilde{A}}^{\cdot }\left(x\right)$ characterizes the extent that the element *x* satisfies to the irrelevant property corresponding to tripolar FS $\tilde{A}$, and $\delta_{\tilde{A}}^{\cdot }\left(x\right)$ characterizes the extent that *x* satisfies to the implicit counter property of TF set $\tilde{A}$. For simplicity, we denote by −*t*=〈*μ*, *λ*, *δ*〉 a TFS and call it a TFN.

**Remark 1 .**

In Definition 3, for a TFS −*t*=〈*μ*, *λ*, *δ*〉, if *δ*=0, then, it reduces to an IFS −*t*=〈*μ*, *λ*〉, and if *λ*=0, it reduces to a BFS, −*t*=〈*μ*, *δ*〉.

In order to rank TFNs, we need to define the score and accuracy functions.

**Definition 4 .**

The score function Ⓢ(−*t*) of a TFN, −*t*=(*μ*, *λ*, *δ*), is defined as follows:

(5) $$\begin{array}{c} Ⓢ\left(-t\right)=\frac{1+\mu +\lambda +\delta }{3},Ⓢ\left(-t\right)\in \left[0,1\right]. \end{array}$$

**Definition 5 .**

The accuracy function *ac*(−*t*) of a TFN −*t*=(*μ*, *λ*, *δ*) is evaluated as follows:

(6) $$\begin{array}{c} ac\left(-t\right)=\frac{\mu -\delta }{2},\;ac\left(-t\right)\in \left[0,\;1\right]. \end{array}$$

Note that *ac*(−*t*) measures the degree of accuracy of −*t*=(*μ*, *λ*, *δ*). Largest value of *ac*(−*t*) shows that the TFN, −*t*=(*μ*, *λ*, *δ*), is more accurate. In the following, we create an ordered relationship between two TFNs, −*t*_1_=(*μ*_1_, *λ*_1_, *δ*_1_) and −*t*_2_=(*μ*_2_, *λ*_2_, *δ*_2_), using *sc*(−*t*) and *ac*(−*t*).

**Definition 6 .**

If Ⓢ(−*t*_1_) ˂ Ⓢ(−*t*_2_) or Ⓢ(−*t*_1_) = Ⓢ(−*t*_2_) but *ac*(−*t*_1_) < *ac*(−*t*_2_), then −*t*_1_ is less than −*t*_2_ referred to as −*t*_1_ < −*t*_2_; if Ⓢ(−*t*_1_)=Ⓢ(−*t*_2_) and *ac*(−*t*_1_) < *ac*(−*t*_2_), then −*t*_1_=−*t*_2_.

The following are some basic TFN operations.

**Definition 7 .**

Let −*t*_*r*_=(*μ*_*r*_, *λ*_*r*_, *δ*_*r*_),  (*r*=1,2), and −*t*=(*μ*, *λ*, *δ*) be any three TFNs and *κ* > 0; then, we have

−*t*_1_ ⊕ −*t*_2_=(*μ*_1_+*μ*_2_ − *μ*_1_*μ*_2_, *λ*_1_*λ*_2_, −|*δ*_1_‖*δ*_2_|).
−*t*_1_ ⊗ −*t*_2_=(*μ*_1_*μ*_2_, *λ*_1_+*λ*_2_ − *λ*_1_*λ*_2_, *δ*_1_+*δ*_2_ − *δ*_1_*δ*_2_).
- *κ*(−*t*)=(1 − (1 − *μ*)^*κ*^, *λ*^*κ*^, −|*δ*|^*κ*^).
- (−*t*)^*κ*^=(*μ*^*κ*^, 1 − (1 − *λ*)^*κ*^, −1+|1+*δ*|^*κ*^).
- (−*t*)^*c*^=(*λ*, *μ*, |*δ*| − 1).
−*t*_1_⊆−*t*_2_ if and only if *μ*_1_ ≤ *μ*_2_, *λ*_1_ ≤ *λ*_2_ and *δ*_1_ ≥ *δ*_2_.
−*t*_1_ ∪ −*t*_2_=(max{*μ*_1_, *μ*_2_},  min{*λ*_1_, *λ*_2_},  min{*δ*_1_, *δ*_2_}).
−*t*_1_ ∪ −*t*_2_=(min{*μ*_1_, *μ*_2_},  max{*λ*_1_, *λ*_2_},  max{*δ*_1_, *δ*_2_}).

We may simply obtain the following operations from Definition 7.

**Theorem 1 .**

Let −*t*_*j*_=(*μ*_*r*_, *λ*_*r*_, *δ*_*r*_),  (*r*=1,2), and −*t*=(*μ*, *λ*, *δ*) be any three TFNs and *κ*, *κ*_1_, *κ*_2_ > 0; then,

−*t*_1_ ⊕ −*t*_2_=−*t*_2_ ⊕ −*t*.
−*t*_1_ ⊗ −*t*_2_=−*t*_2_ ⊗ −*t*_1_.
3. *κ*(−*t*_1_ ⊕ −*t*_2_)=*κ*(−*t*_1_) ⊕ *κ*(−*t*_2_).
4. (−*t*_1_ ⊗ −*t*_2_)^*κ*^=(−*t*_1_)^*κ*^ ⊗ (−*t*_2_)^*κ*^.
5. *κ*_1_ − *t* ⊕ *κ*_2_ − *t*=(*κ*_1_+*κ*_2_) − *t*.
6. (−*t*)^*κ*_1_^ ⊗ (−*t*)^*κ*_2_^=(−*t*)^*κ*_1_+*κ*_2_^.
7. ((−*t*)^*κ*_1_^)^*κ*_2_^=(−*t*)^*κ*_1_*κ*_2_^.

Dombi product and Dombi sum are special cases of triangle norms and conorms, which are defined further below.

**Definition 8 (Dombi [38]).**

Assume that *α* and *β* can be any two real numbers. The following formulas define Dombi *T*-norms and *T*-conorms.

(7) $$\begin{array}{c} \text{Dombi}\left(\alpha ,\beta \right)=\frac{1}{1+{\left\{{\left(1-\alpha /\alpha \right)}^{ℜ}+{\left(1-\beta /\beta \right)}^{ℜ}\right\}}^{\left(1/ℜ\right)}}, \end{array}$$

(8) $$\begin{array}{c} {\text{Dombi}}^{c}\left(\alpha ,\beta \right)=1-\frac{1}{1+{\left\{{\left(\alpha /1-\alpha \right)}^{ℜ}+{\left(\beta /1-\beta \right)}^{ℜ}\right\}}^{\left(1/ℜ\right)}}, \end{array}$$

where *ℜ* ≥ 1 and (*α*, *β*) ∈ [0,1] × [0,1].

### 2.1. TF-Dombi Operations

In light of DTN and DTCN, we use TFNs to clarify Dombi operations in this section. On the basis of Dombi operations, we will suggest some TFN operating laws.

**Definition 9 .**

Let −*t*_*r*_=(*μ*_*r*_, *λ*_*r*_, *δ*_*r*_),  (*r*=1,2), be TFNs and *ℜ* ≥ 1 and *κ* > 0; then, the D *T*-norm and *T*-conorm operations of TFNs are introduced as follows:

$-t_{1}⊕-t_{2}=\left(\begin{array}{c} 1-\left(1/1+{\left\{{\left(\mu_{1}/1-\mu_{1}\right)}^{ℜ}+{\left(\mu_{2}/1-\mu_{2}\right)}^{ℜ}\right\}}^{\left(1/ℜ\right)}\right),\left(1/1+{\left\{{\left(1-\lambda_{1}/\lambda_{1}\right)}^{ℜ}+{\left(1-\lambda_{2}/\lambda_{2}\right)}^{ℜ}\right\}}^{\left(1/ℜ\right)}\right),\\ \left(-1/1+{\left\{{\left(\delta_{1}+1/\left|\delta_{1}\right|\right)}^{ℜ}+{\left(\delta_{2}+1/\left|\delta_{2}\right|\right)}^{ℜ}\right\}}^{\left(1/ℜ\right)}\right) \end{array}\right)$.
$-t_{1}⊗-t_{2}=\left(\begin{array}{c} \left(1/1+{\left\{{\left(1-\mu_{1}/\mu_{1}\right)}^{ℜ}+{\left(1-\mu_{2}/\mu_{2}\right)}^{ℜ}\right\}}^{\left(1/ℜ\right)}\right),1-\left(1/1+{\left\{{\left(\lambda_{1}/1-\lambda_{1}\right)}^{ℜ}+{\left(\lambda_{2}/1-\lambda_{2}\right)}^{ℜ}\right\}}^{\left(1/ℜ\right)}\right),\\ -1+\left(1/1+{\left\{{\left(\left|\delta_{1}\right|/\delta_{1}+1\right)}^{ℜ}+{\left(\left|\delta_{2}\right|/\delta_{2}+1\right)}^{ℜ}\right\}}^{\left(1/ℜ\right)}\right) \end{array}\right)$.
- $\kappa \left(-t_{1}\right)=\left(\begin{array}{c} 1-\left(1/1+{\left\{\kappa {\left(\mu_{1}/1-\mu_{1}\right)}^{ℜ}\right\}}^{\left(1/ℜ\right)}\right),\left(1/1+{\left\{\kappa {\left(1-\lambda_{1}/\lambda_{1}\right)}^{ℜ}\right\}}^{\left(1/ℜ\right)}\right),\\ \left(-1/1+{\left\{\kappa {\left(\delta_{1}+1/\left|\delta_{1}\right|\right)}^{ℜ}\right\}}^{\left(1/ℜ\right)}\right) \end{array}\right)$.
${\left(-t_{1}\right)}^{\kappa }=\left(\begin{array}{c} \left(1/1+{\left\{\kappa {\left(1-\mu_{1}/\mu_{1}\right)}^{ℜ}\right\}}^{\left(1/ℜ\right)}\right),1-\left(1/1+{\left\{\kappa {\left(\lambda_{1}/1-\lambda_{1}\right)}^{ℜ}\right\}}^{\left(1/ℜ\right)}\right),\\ -1+\left(1/1+{\left\{\kappa {\left(\left|\delta_{1}\right|/\delta_{1}+1\right)}^{ℜ}\right\}}^{\left(1/ℜ\right)}\right) \end{array}\right)$.

### 2.2. TF Dombi Averaging AOs

In this section, we create and examine the basic features of the TF-Dombi weighted averaging (TFDWA) operator, TF-Dombi ordered weighted averaging (TFDOWA) operator, and TF-Dombi hybrid weight averaging (TFDHWA) operator, which are all arithmetic aggregation operators using TFNs.

**Definition 10 .**

Let −*t*_*r*_=(*μ*_*r*_, *λ*_*r*_, *δ*_*r*_),  (*r*=1,…, *p*), be a collection of TFNs. Then, the TF-Dombi TFDWA operator is a mapping TFDWA:−*t*^*n*^⟶−*t* such that

(9) $$\begin{array}{c} {\text{TFDWA}}_{\Phi }\left(-t_{1},-t_{2},\ldots ,-t_{p}\right)=\overset{p}{\underset{r=1}{⊕}}\left(\Phi_{r}-t_{r}\right), \end{array}$$

where Φ=(Φ_1_, Φ_2_,…,Φ_*p*_)^*T*^ is the weight vector of −*t*_*r*_,  (*r*=1,…, *p*) with the conditions Φ_*r*_ > 0 and ⊕_*r*=1_^*p*^Φ_*r*_=1.

**Remark 2 .**

In Definition 10, the collection of TFNs −*t*_*r*_=(*μ*_*r*_, *λ*_*r*_, *δ*_*r*_),  (*r*=1,…, *p*), we have

- If *δ*_*r*_=0, for all *r*, 1 ≤ *r* ≤ *p*, then the family of TFNs, −*t*_*r*_,  (*r*=1,…, *p*), reduces to a family of IFNs, −*t*_*r*_=(*μ*_*r*_, *λ*_*r*_),  (*r*=1,…, *p*).
- If *λ*_*r*_=0, for all *r*, 1 ≤ *r* ≤ *p*, then the family of TFNs, −*t*_*r*_,  (*r*=1,…, *p*), reduces to a family of BFNs, −*t*_*r*_=(*μ*_*r*_, *δ*_*r*_),  (*r*=1,…, *p*).

In the theorem mentioned below, we use the Dombi operation on TFNs and develop TFDWA operator for the aggregation of TFNs.

**Theorem 2 .**

Let −*t*_*r*_=(*μ*_*r*_, *λ*_*r*_, *δ*_*r*_),  (*r*=1,…, *p*), be a family of TFNs; then, the aggregated value of this family by using the TFDWA operator is also a TFN, and

(10) $$\begin{array}{c} {\text{TFDWA}}_{\Phi }\left(-t_{1},-t_{2},\ldots ,-t_{p}\right)\\ =\overset{p}{\underset{r=1}{⊕}}\left(\Phi_{r}-t_{r}\right)=\left(\begin{array}{c} 1-\frac{1}{1+{\left\{{⊕}_{r=1}^{p}\Phi_{r}{\left(\mu_{r}/1-\mu_{r}\right)}^{ℜ}\right\}}^{\left(1/ℜ\right)}},\frac{1}{1+{\left\{{⊕}_{r=1}^{p}\Phi_{r}{\left(1-\lambda_{r}/\lambda_{r}\right)}^{ℜ}\right\}}^{\left(1/ℜ\right)}},\\ \frac{-1}{1+{\left\{{⊕}_{r=1}^{p}\Phi_{r}{\left(1+\delta_{r}/\left|\delta_{r}\right|\right)}^{ℜ}\right\}}^{\left(1/ℜ\right)}} \end{array}\right), \end{array}$$

where Φ=(Φ_1_, Φ_2_,…,Φ_*p*_)^*T*^ is the weight vector of −*t*_*r*_,  (*r*=1,…, *p*) with Φ_*r*_ > 0 and ⊕_*r*=1_^*p*^Φ_*r*_=1.

**Proof**

The mathematical induction approach can be used to prove this theorem. Thus,

(i) When *p*=2, based on TFNs' Dombi operation, as defined in Definition 9, we obtain
  (11) $$\begin{array}{c} {\text{TFDWA}}_{\Phi }\left(-t_{1},-t_{2}\right)=\Phi_{1}-t_{1}⊕\Phi_{2}-t_{2}=\Phi_{1}\left(\mu_{1},\lambda_{1},\delta_{1}\right)⊕\Phi_{2}\left(\mu_{2},\lambda_{2},\delta_{2}\right). \end{array}$$
For the RHS of equation (10), we have
  (12) $$\begin{array}{c} \left(\begin{array}{c} 1-\frac{1}{1+{\left\{\Phi_{1}{\left(\mu_{1}/1-\mu_{1}\right)}^{ℜ}+\Phi_{2}{\left(\mu_{2}/1-\mu_{2}\right)}^{ℜ}\right\}}^{\left(1/ℜ\right)}},\frac{1}{1+{\left\{\Phi_{1}{\left(1-\lambda_{1}/\lambda_{1}\right)}^{ℜ}+\Phi_{2}{\left(1-\lambda_{2}/\lambda_{2}\right)}^{ℜ}\right\}}^{\left(1/ℜ\right)}},\\ \frac{-1}{1+{\left\{\Phi_{1}{\left(1+\delta_{1}/\left|\delta_{1}\right|\right)}^{ℜ}+\Phi_{2}{\left(1+\delta_{2}/\left|\delta_{2}\right|\right)}^{ℜ}\right\}}^{\left(1/ℜ\right)}} \end{array}\right)\\ =\left(\begin{array}{c} 1-\frac{1}{1+{\left\{\sum_{r=1}^{2}\Phi_{r}{\left(\mu_{r}/1-\mu_{r}\right)}^{ℜ}\right\}}^{\left(1/ℜ\right)}},\frac{1}{1+{\left\{\sum_{r=1}^{2}\Phi_{r}{\left(1-\lambda_{r}/\lambda_{r}\right)}^{ℜ}\right\}}^{\left(1/ℜ\right)}},\\ \frac{-1}{1+{\left\{\sum_{r=1}^{2}\Phi_{r}{\left(1+\delta_{r}/\left|\delta_{r}\right|\right)}^{ℜ}\right\}}^{\left(1/ℜ\right)}} \end{array}\right). \end{array}$$
Thus, equation (9) holds for *p*=2.
(ii) Assume that equation (9) holds for *p*=*k*, where *k* ∈ *ℕ*(set of natural numbers); then, equation (9) becomes
  (13) $$\begin{array}{c} {\text{TFDWA}}_{\Phi }\left({ŧ}_{1},{ŧ}_{2},\ldots ,{ŧ}_{k}\right)\\ =\overset{k}{\underset{r=1}{⊕}}\left(\Phi_{r}-t_{r}\right)=\left(\begin{array}{c} 1-\frac{1}{1+{\left\{\sum_{r=1}^{k}\Phi_{r}{\left(\mu_{r}/1-\mu_{r}\right)}^{ℜ}\right\}}^{\left(1/ℜ\right)}},\frac{1}{1+{\left\{\sum_{r=1}^{k}\Phi_{r}{\left(1-\lambda_{r}/\lambda_{r}\right)}^{ℜ}\right\}}^{\left(1/ℜ\right)}},\\ \frac{-1}{1+{\left\{\sum_{r=1}^{k}\Phi_{r}{\left(1+\delta_{r}/\left|\delta_{r}\right|\right)}^{ℜ}\right\}}^{\left(1/ℜ\right)}} \end{array}\right). \end{array}$$
Now for *p*=*k*+1, we have the following equation.
  (14) $$\begin{array}{c} {\text{TFDWA}}_{\Phi }\left(-t_{1},-t_{2},\ldots ,-t_{k},-t_{k+1}\right)\\ =\overset{k}{\underset{r=1}{⊕}}\left(\Phi_{r}-t_{r}\right)⊕\left(\Phi_{k+1}-t_{k+1}\right)\\ =\left(\begin{array}{c} 1-\frac{1}{1+{\left\{\sum_{r=1}^{k}\Phi_{r}{\left(\mu_{r}/1-\mu_{r}\right)}^{ℜ}\right\}}^{\left(1/ℜ\right)}},\frac{1}{1+{\left\{\sum_{r=1}^{k}\Phi_{r}{\left(1-\lambda_{r}/\lambda_{r}\right)}^{ℜ}\right\}}^{\left(1/ℜ\right)}},\\ \frac{-1}{1+{\left\{\sum_{r=1}^{k}\Phi_{r}{\left(1+\delta_{r}/\left|\delta_{r}\right|\right)}^{ℜ}\right\}}^{\left(1/ℜ\right)}} \end{array}\right)\\ ⊕\left(\begin{array}{c} 1-\frac{1}{1+{\left\{\Phi_{k+1}{\left(\mu_{k+1}/1-\mu_{k+1}\right)}^{ℜ}\right\}}^{\left(1/ℜ\right)}},\frac{1}{1+{\left\{\Phi_{k+1}{\left(1-\lambda_{k+1}/\lambda_{k+1}\right)}^{ℜ}\right\}}^{\left(1/ℜ\right)}},\\ \frac{-1}{1+{\left\{\Phi_{k+1}{\left(1+\delta_{k+1}/\left|\delta_{k+1}\right|\right)}^{ℜ}\right\}}^{\left(1/ℜ\right)}} \end{array}\right)\\ =\left(\begin{array}{c} 1-\frac{1}{1+{\left\{\sum_{r=1}^{k+1}\Phi_{r}{\left(\mu_{r}/1-\mu_{r}\right)}^{ℜ}\right\}}^{\left(1/ℜ\right)}},\frac{1}{1+{\left\{\sum_{r=1}^{k+1}\Phi_{r}{\left(1-\lambda_{r}/\lambda_{r}\right)}^{ℜ}\right\}}^{\left(1/ℜ\right)}},\\ \frac{-1}{1+{\left\{\sum_{r=1}^{k+1}\Phi_{r}{\left(1+\delta_{r}/\left|\delta_{r}\right|\right)}^{ℜ}\right\}}^{\left(1/ℜ\right)}}. \end{array}\right) \end{array}$$
Thus, equation (9) is true for *p*=*k*+1. Therefore, equation (9) is true for any *p* ∈ *ℕ*.

**Remark 3 .**

In Theorem 2, as part of a collection of TFNs, −*t*_*r*_=(*μ*_*r*_, *λ*_*r*_, *δ*_*r*_),  (*r*=1,…, *p*), if

(i) *δ*_*r*_=0, for all *r*, then the collection of TFNs, −*t*_*r*_=(*μ*_*r*_, *λ*_*r*_, *δ*_*r*_), becomes a collection of IFNs, −*t*_*r*_=(*μ*_*r*_, *λ*_*r*_),  (*r*=1,…, *p*), and the TFDWA operator reduces to the IFDWA operator, as shown below.
  (15) $$\begin{array}{c} {\text{IFDWA}}_{\Phi }\left(-t_{1},-t_{2},\ldots ,-t_{p}\right)\\ =\overset{p}{\underset{r=1}{⊕}}\left(\Phi_{r}-t_{r}\right)=\left(1-\frac{1}{1+{\left\{{⊕}_{r=1}^{p}\Phi_{r}{\left(\mu_{r}/1-\mu_{r}\right)}^{ℜ}\right\}}^{\left(1/ℜ\right)}},\frac{1}{1+{\left\{{⊕}_{r=1}^{p}\Phi_{r}{\left(1-\lambda_{r}/\lambda_{r}\right)}^{ℜ}\right\}}^{\left(1/ℜ\right)}}\right). \end{array}$$
(ii) If *λ*_*r*_=0, for all *r*, then the collection of TFNs, −*t*_*r*_=(*μ*_*r*_, *λ*_*r*_, *δ*_*r*_), becomes a collection of BFNs, −*t*_*r*_=(*μ*_*r*_, *δ*_*r*_),  (*r*=1,…, *p*), and the TFDWA operator reduces to the BFDWA operator, as given below.
  (16) $$\begin{array}{c} {\text{BFDWA}}_{\Phi }\left(-t_{1},-t_{2},\ldots ,-t_{p}\right)\\ =\overset{p}{\underset{r=1}{⊕}}\left(\Phi_{r}-t_{r}\right)=\left(1-\frac{1}{1+{\left\{{⊕}_{r=1}^{p}\Phi_{r}{\left(\mu_{r}/1-\mu_{r}\right)}^{ℜ}\right\}}^{\left(1/ℜ\right)}},\frac{-1}{1+{\left\{{⊕}_{r=1}^{p}\Phi_{r}{\left(1+\delta_{r}/\left|\delta_{r}\right|\right)}^{ℜ}\right\}}^{\left(1/ℜ\right)}}\right). \end{array}$$

The TFDWA operator has a number of essential qualities, which are given below.

**Theorem 3 (idempotency property).**

If −*t*_*r*_=(*μ*_*r*_, *λ*_*r*_, *δ*_*r*_),  (*r*=1,…, *p*), is a set of TFNs that all have the same value, i.e., if −*t*_*r*_=(*μ*_*r*_, *λ*_*r*_, *δ*_*r*_) = −*t*=(*μ*, *λ*, *δ*) for all *r*, then

(17) $$\begin{array}{c} {\text{TFDWA}}_{\Phi }\left(-t_{1},-t_{2},\ldots ,-t_{r}\right)=-t. \end{array}$$

**Proof**

Since −*t*_*r*_=(*μ*_*r*_, *λ*_*r*_, *δ*_*r*_) = −*t*(*r*=1,…, *p*), then by using equation (9), we have

(18) $$\begin{array}{c} {\text{TFDWA}}_{\Phi }\left(-t_{1},-t_{2},\ldots ,-t_{r}\right)\\ =\overset{p}{\underset{r=1}{⊕}}\left(\Phi_{r}-t_{r}\right)=\left(\begin{array}{c} 1-\frac{1}{1+{\left\{{⊕}_{r=1}^{p}\Phi_{r}{\left(\mu_{r}/1-\mu_{r}\right)}^{ℜ}\right\}}^{\left(1/ℜ\right)}},\frac{1}{1+{\left\{{⊕}_{r=1}^{p}\Phi_{r}{\left(1-\lambda_{r}/\lambda_{r}\right)}^{ℜ}\right\}}^{\left(1/ℜ\right)}},\\ \frac{-1}{1+{\left\{{⊕}_{r=1}^{p}\Phi_{r}{\left(1+\delta_{r}/\left|\delta_{r}\right|\right)}^{ℜ}\right\}}^{\left(1/ℜ\right)}} \end{array}\right)\\ =\left(1-\frac{1}{1+{\left\{{\left(\mu /1-\mu \right)}^{ℜ}\right\}}^{\left(1/ℜ\right)}},\frac{1}{1+{\left\{{\left(1-\lambda /\lambda \right)}^{ℜ}\right\}}^{\left(1/ℜ\right)}},\frac{-1}{1+{\left\{{\left(1+\delta /\left|\delta \right|\right)}^{ℜ}\right\}}^{\left(1/ℜ\right)}}\right)\\ =\left(1-\frac{1}{1+\left(\mu /1-\mu \right)},\frac{1}{1+\left(1-\lambda /\lambda \right)},\frac{-1}{1+\left(1+\delta /\left|\delta \right|\right)}\right)=\left(\mu ,\lambda ,\delta \right). \end{array}$$

Thus, TFDWA_Φ_(−*t*_1_, −*t*_2_,…, −*t*_*r*_)=*t*.

In a similar manner, we can verify the following properties of the TFDWA operator.

**Theorem 4 (boundedness property).**

Let −*t*_*r*_=(*μ*_*r*_, *λ*_*r*_, *δ*_*r*_),  (*r*=1,2,…, *p*), be a family of TFNs, and −*t*^−^ = min{−*t*_*r*_} and −*t*^+^ = max{−*t*_*r*_}. Then,

(19) $$\begin{array}{c} -t^{-}\leq {\text{TFDWA}}_{\Phi }\left(-t_{1},-t_{2},\ldots ,-t_{p}\right)\leq -t^{+}. \end{array}$$

**Theorem 5 (monotonicity property).**

If −*t*_*r*_=(*μ*_*r*_, *λ*_*r*_, *δ*_*r*_),  (*r*=1,…, *p*), and −*t*_*r*_′=(*μ*_*r*_′, *λ*_*r*_′, *δ*_*r*_′),  (*r*=1,2,…, *p*), are the families of TFNs, such that −*t*_*r*_ ≤ −*t*_*r*_′ for all *r*, then

(20) $$\begin{array}{c} {\text{TFDWA}}_{\Phi }\left(-t_{1},-t_{2},\ldots ,-t_{p}\right)\leq {\text{TFDWA}}_{\Phi }\left(-t_{1}^{\prime },-t_{2}^{\prime },\ldots ,-t_{p}^{\prime }\right). \end{array}$$

Now we will go through the fundamental features of the TFDOWA operator.

**Definition 11 .**

Let −*t*_*r*_=(*μ*_*r*_, *λ*_*r*_, *δ*_*r*_),  (*r*=1,…, *p*), be a collection of TFNs. A TFDOWA operator of dimension *p* is a mapping TFDOWA:−*t*^*p*^⟶*t* with an associated weight vector *ω*=(*ω*_1_, *ω*_2_,…,*ω*_*p*_)^*T*^ such that *ω*_*r*_ > 0, and ⊕_*r*=1_^*p*^*ω*_*r*_=1. Therefore,

(21) $$\begin{array}{c} {\text{TFDOWA}}_{\Phi }\left(-t_{1},-t_{2},\ldots ,-t_{p}\right)={⊕}_{r=1}^{p}\left(\Phi_{r}-t_{r\left(\sigma \right)}\right), \end{array}$$

where (*σ*(1), *σ*(2),…, *σ*(*p*)) are the permutations of *σ*(*r*) (*r*=1,2,…, *p*) for which −*t*_*σ*(*r* − 1)_ ≥ −*t*_*σ*(*r*)_ for all *r*=1,2,…, *p*.

The following theorem is a consequence of Definition 10 and Theorem 2.

**Theorem 6 .**

Let −*t*_*r*_=(*μ*_*r*_, *λ*_*r*_, *δ*_*r*_),  (*r*=1,…, *p*), be a family of TFNs. A TFDOWA operator of dimension *p* is a mapping from −*t*^*p*^ to *t* with the associated weight vector *ω*=(*ω*_1_, *ω*_2_,…,*ω*_*p*_)^*T*^ such that *ω*_*r*_ > 0 and ⊕_*r*=1_^*p*^*ω*_*r*_=1. Then,

(22) $$\begin{array}{c} {\text{TFDOWA}}_{\omega }\left(-t_{1},-t_{2},\ldots ,-t_{p}\right)\\ ={⊕}_{r=1}^{p}\left(\Phi_{r}-t_{r\left(\sigma \right)}\right)=\left(\begin{array}{c} 1-\frac{1}{1+{\left\{{⊕}_{r=1}^{p}\omega_{r}{\left(\mu_{\sigma \left(r\right)}/1-\mu_{\sigma \left(r\right)}\right)}^{ℜ}\right\}}^{\left(1/ℜ\right)}},\frac{1}{1+{\left\{{⊕}_{r=1}^{p}\omega_{r}{\left(1-\lambda_{\sigma \left(r\right)}/\lambda_{\sigma \left(r\right)}\right)}^{ℜ}\right\}}^{\left(1/ℜ\right)}},\\ \frac{1}{1+{\left\{{⊕}_{r=1}^{p}\omega_{r}{\left(1+\delta_{\sigma \left(r\right)}/\left|\delta_{\sigma \left(r\right)}\right|\right)}^{ℜ}\right\}}^{\left(1/ℜ\right)}} \end{array}\right), \end{array}$$

where (*σ*(1), *σ*(2),…, *σ*(*p*)) are the permutations of *σ*(*r*) (*r*=1,2,…, *p*) for which −*t*_*σ*(*r* − 1)_ ≥ −*t*_*σ*(*r*)_ for all *r*=1,2,…, *p*.

**Remark 4 .**

In Definition 10, the collection of TFNs −*t*_*r*_=(*μ*_*r*_, *λ*_*r*_, *δ*_*r*_),  (*r*=1,…, *p*), we have

(i) If *δ*_*r*_=0, for all *r*, then the TFDOWA operator decreases to IFDOWA operator and
  (23) $$\begin{array}{c} {\text{IFDOWA}}_{\omega }\left(-t_{1},-t_{2},\ldots ,-t_{p}\right)\\ ={⊕}_{r=1}^{p}\left(\Phi_{r}-t_{r\left(\sigma \right)}\right)=\left(1-\frac{1}{1+{\left\{{⊕}_{r=1}^{p}\omega_{r}{\left(\mu_{\sigma \left(r\right)}/1-\mu_{\sigma \left(r\right)}\right)}^{ℜ}\right\}}^{\left(1/ℜ\right)}},\frac{1}{1+{\left\{{⊕}_{r=1}^{p}\omega_{r}{\left(1-\lambda_{\sigma \left(r\right)}/\lambda_{\sigma \left(r\right)}\right)}^{ℜ}\right\}}^{\left(1/ℜ\right)}}\right). \end{array}$$
(ii) If *λ*_*r*_=0, for all *r*, then the TFDOWA operator decreases to BFDOWA operator and
  (24) $$\begin{array}{c} {\text{BFDOWA}}_{\omega }\left(-t_{1},-t_{2},\ldots ,-t_{p}\right)\\ ={⊕}_{r=1}^{p}\left(\Phi_{r}-t_{r\left(\sigma \right)}\right)=\left(1-\frac{1}{1+{\left\{{⊕}_{r=1}^{p}\omega_{r}{\left(\mu_{\sigma \left(r\right)}/1-\mu_{\sigma \left(r\right)}\right)}^{ℜ}\right\}}^{\left(1/ℜ\right)}},\frac{1}{1+{\left\{{⊕}_{r=1}^{p}\omega_{r}{\left(1+\delta_{\sigma \left(r\right)}/\left|\delta_{\sigma \left(r\right)}\right|\right)}^{ℜ}\right\}}^{\left(1/ℜ\right)}}\right). \end{array}$$

The following properties of a TFDOWA operator can easily be proved.

(P1) (idempotency property). If −*t*_*r*_=(*μ*_*r*_, *λ*_*r*_, *δ*_*r*_) (*r*=1,2,…, *p*) are all equal, i.e., −*t*_*r*_=−*t* for all *r*, then TFDOWA_*ω*_(−*t*_1_, −*t*_2_,…, −*t*_*p*_)=*t*.
(P2) (boundedness property). Let −*t*_*r*_=(*μ*_*r*_, *λ*_*r*_, *δ*_*r*_), (*r*=1,2,…, *p*), be a family of TFNs and −*t*^−^ = min − *t*_*r*_ and −*t*^+^ = max − *t*_*r*_. Then,
  (25) $$\begin{array}{c} -t^{-}\leq {\text{TFDOWA}}_{\omega }\left(-t_{1},-t_{2},\ldots ,-t_{p}\right)\leq -t^{+}. \end{array}$$
(P3) (monotonicity property). If −*t*_*r*_=(*μ*_*r*_, *λ*_*r*_, *δ*_*r*_), (*r*=1,2,…, *p*), and −*t*_*r*_′=(*μ*_*r*_′, *λ*_*r*_′, *δ*_*r*_′),  (*r*=1,2,…, *p*), are two TFNs such that −*t*_*r*_ ≤ −*t*_*r*_′ for all *r*, then
  (26) $$\begin{array}{c} {\text{TFDOWA}}_{\omega }\left(-t_{1},-t_{2},\ldots ,-t_{p}\right)\leq {\text{TFDOWA}}_{\omega }\left(-t_{1}^{\prime },-t_{2}^{\prime },\ldots ,-t_{p}^{\prime }\right). \end{array}$$

**Definition 12 .**

A TFDHWA operator of dimension *p* is a mapping TFDHA:−*t*^*p*^⟶*t* with the associated weight vector *w*=(*w*_1_, *w*_2_,…, *w*_*p*_) such that *w*_*r*_ > 0 and ⊕_*r*=1_^*p*^*w*_*r*_=1 and the TFDHWA operator is provided by the following equation:

(27) $$\begin{array}{c} {\text{TFDHWA}}_{\left(w,\Phi \right)}\left(-t_{1},-t_{2},\ldots ,-t_{p}\right)\\ =\left(\left(w_{1}-t_{\sigma \left(1\right)}^{\cdot }\right),\left(w_{2}-t_{\sigma \left(2\right)}^{\cdot }\right),\ldots ,\left(w_{p}-t_{\sigma \left(p\right)}^{\cdot }\right)\right)\\ =\left(\begin{array}{c} 1-\frac{1}{1+{\left\{{⊕}_{r=1}^{p}w_{r}{\left(\mu_{\sigma \left(r\right)}^{\cdot }/1-\mu_{\sigma \left(r\right)}^{\cdot }\right)}^{ℜ}\right\}}^{\left(1/ℜ\right)}},\frac{1}{1+{\left\{{⊕}_{r=1}^{p}w_{r}{\left(1-\lambda_{\sigma \left(r\right)}^{\cdot }/\lambda_{\sigma \left(r\right)}^{\cdot }\right)}^{ℜ}\right\}}^{\left(1/ℜ\right)}},\\ \frac{1}{1+{\left\{{⊕}_{r=1}^{p}w_{r}{\left(1+\delta_{\sigma \left(r\right)}^{\cdot }/\left|\delta_{\sigma \left(r\right)}^{\cdot }\right|\right)}^{ℜ}\right\}}^{\left(1/ℜ\right)}} \end{array}\right), \end{array}$$

where −*t*_*σ*(*r*)_^·^ is the *r*^th^ largest WTF number −*t*_*r*_^·^,  (−*t*_*r*_^·^=*p*Φ_*r*_ − *t*_*r*_,  *r*=1,2,…, *p*) and Φ=(Φ_1_, Φ_2_,…,Φ_*p*_)^*T*^ is the weight vector of −*t*_*r*_^·^ with the condition Φ_*r*_ > 0 and ⊕_*r*=1_^*p*^Φ_*r*_=1, where *p* is the balancing coefficient. Some important properties of (TFDHWA) operator are given below:

- When *w*=((1/*p*), (1/*p*),…, (1/*p*)), then TFDWA operator is a special case of TFDHA operator.
- When, Φ=((1/*p*), (1/*p*),…, (1/*p*)), then TFDOWA operator is a special case of the TFDHWA operator. As a result, we conclude that the TFDHWA operator is a generalization of both the TFDWA and TFDOWA operators.

**Remark 5 .**

In Definition 12, the collection of TFNs −*t*_*r*_=(*μ*_*r*_, *λ*_*r*_, *δ*_*r*_),  (*r*=1,…, *p*), we have

(i) If *δ*_*r*_=0, for all *r*, then the TFDHWA operator reduces to IFDHWA operator and
  (28) $$\begin{array}{c} {\text{IFDHWA}}_{\left(w,\Phi \right)}\left(-t_{1},-t_{2},\ldots ,-t_{p}\right)\\ =\left(\left(w_{1}-t_{\sigma \left(1\right)}^{\cdot }\right),\left(w_{2}-t_{\sigma \left(2\right)}^{\cdot }\right),\ldots ,\left(w_{p}-t_{\sigma \left(p\right)}^{\cdot }\right)\right)\\ =\left(1-\frac{1}{1+{\left\{{⊕}_{r=1}^{p}w_{r}{\left(\mu_{\sigma \left(r\right)}^{\cdot }/1-\mu_{\sigma \left(r\right)}^{\cdot }\right)}^{ℜ}\right\}}^{\left(1/ℜ\right)}},\frac{1}{1+{\left\{{⊕}_{r=1}^{p}w_{r}{\left(1-\lambda_{\sigma \left(r\right)}^{\cdot }/\lambda_{\sigma \left(r\right)}^{\cdot }\right)}^{ℜ}\right\}}^{\left(1/ℜ\right)}}\right). \end{array}$$
(ii) If *λ*_*r*_=0, for all *r*, then the TFDHWA operator reduces to BFDHWA operator and
  (29) $$\begin{array}{c} {\text{BFDHWA}}_{\left(w,\Phi \right)}\left(-t_{1},-t_{2},\ldots ,-t_{p}\right)\\ =\left(\left(w_{1}-t_{\sigma \left(1\right)}^{\cdot }\right),\left(w_{2}-t_{\sigma \left(2\right)}^{\cdot }\right),\ldots ,\left(w_{p}-t_{\sigma \left(p\right)}^{\cdot }\right)\right)\\ =\left(1-\frac{1}{1+{\left\{{⊕}_{r=1}^{p}w_{r}{\left(\mu_{\sigma \left(r\right)}^{\cdot }/1-\mu_{\sigma \left(r\right)}^{\cdot }\right)}^{ℜ}\right\}}^{\left(1/ℜ\right)}},\frac{1}{1+{\left\{{⊕}_{r=1}^{p}w_{r}{\left(1+\delta_{\sigma \left(r\right)}^{\cdot }/\left|\delta_{\sigma \left(r\right)}^{\cdot }\right|\right)}^{ℜ}\right\}}^{\left(1/ℜ\right)}}\right). \end{array}$$

We now, give an illustrative example for the verification of Definition 13.

**Example 1 .**

Consider four TFNs, −*t*_1_=(0.5, 0.4, −0.3), −*t*_2_=(0.6, 0.4, −0.3), −*t*_3_=(0.7, 0.2, −0.3), and −*t*_4_=(0.2, 0.4, −0.4), and let Φ=(0.20, 0.30, 0.30, 0.20)^*T*^ be the associated weight vector. Then, by Definition 13, the aggregated value of TFNs for *ℜ*=3, and by using the TFDHWA operator, we get

(30) $$\begin{array}{c} -t_{1}^{\cdot }=\left(\begin{array}{c} 1-\frac{1}{1+{\left\{4\times 0.20{\left(0.5/1-0.5\right)}^{3}\right\}}^{\left(1/3\right)}},\frac{1}{1+{\left\{4\times 0.20{\left(1-0.4/0.4\right)}^{3}\right\}}^{\left(1/3\right)}},\\ \frac{-1}{1+{\left\{4\times 0.20{\left(1-0.3/0.3\right)}^{3}\right\}}^{\left(1/3\right)}} \end{array}\right)\\ =\left(0.4814,0.4179,-0.3158\right)\\ -t_{2}^{\cdot }=\left(\begin{array}{c} 1-\frac{1}{1+{\left\{4\times 0.30{\left(0.6/1-0.6\right)}^{3}\right\}}^{\left(1/3\right)}},\frac{1}{1+{\left\{4\times 0.30{\left(1-0.4/0.4\right)}^{3}\right\}}^{\left(1/3\right)}},\\ \frac{-1}{1+{\left\{4\times 0.30{\left(1-0.3/0.3\right)}^{3}\right\}}^{\left(1/3\right)}} \end{array}\right)\\ =\left(0.6144,0.3855,-0.2873\right)\\ -t_{3}^{\cdot }=\left(\begin{array}{c} 1-\frac{1}{1+{\left\{4\times 0.30{\left(0.7/1-0.7\right)}^{3}\right\}}^{\left(1/3\right)}},\frac{1}{1+{\left\{4\times 0.30{\left(1-0.2/0.2\right)}^{3}\right\}}^{\left(1/3\right)}},\\ \frac{-1}{1+{\left\{4\times 0.30{\left(1-0.3/0.3\right)}^{3}\right\}}^{\left(1/3\right)}} \end{array}\right)\\ =\left(0.7126,0.1904,-0.2874\right)\\ -t_{4}^{\cdot }=\left(\begin{array}{c} 1-\frac{1}{1+{\left\{4\times 0.20{\left(0.2/1-0.2\right)}^{3}\right\}}^{\left(1/3\right)}},\frac{1}{1+{\left\{4\times 0.20{\left(1-0.4/0.4\right)}^{3}\right\}}^{\left(1/3\right)}},\\ \frac{-1}{1+{\left\{4\times 0.20{\left(1-0.4/0.4\right)}^{3}\right\}}^{\left(1/3\right)}} \end{array}\right)\\ =\left(0.1883,0.4179,-0.4179\right). \end{array}$$

Scores of −*t*_*r*_^·^,  (*r*=1,2,3,4) are calculated as follows:

Ⓢ(−*t*_1_^·^)=(1+0.4814+0.4179 − 0.3158/3)=0.5278, Ⓢ(−*t*_2_^·^)=(1+0.6144+0.3855 − 0.2873/3)=0.5708,  Ⓢ(−*t*_3_^·^)=(1+0.7126+0.1904 − 0.2874/3)=0.5385, Ⓢ(−*t*_4_^·^)=(1+0.1883+0.3179 − 0.4179/3)=0.3961.

Since Ⓢ(−*t*_2_^·^) > Ⓢ(−*t*_3_^·^) > Ⓢ(−*t*_1_^·^) > Ⓢ(−*t*_4_^·^), then −*t*_*σ*(1)_^·^ = −*t*_2_^·^=(0.6145, 0.3855, −0.3158), −*t*_*σ*(2)_^·^=−*t*_3_^·^=(0.7126, 0.1904, −0.2874), −*t*_*σ*(3)_^·^ = −*t*_1_^·^=(0.6145, 0.3179, −0.2874), and −*t*_*σ*(4)_^·^ = −*t*_4_^·^=(0.1884, 0.3419, −0.4180). Therefore, by using TFDHWA operator for *ℜ*=3, we get

(31) $$\begin{array}{c} \text{TFDHWA}\left(-t_{\sigma \left(1\right)}^{\cdot },-t_{\sigma \left(2\right)}^{\cdot },\ldots ,-t_{\sigma \left(4\right)}^{\cdot }\right)\\ ={⊕}_{r=1}^{4}\left(\Phi_{r}-t_{\sigma \left(r\right)}^{\cdot }\right)\\ =\left(\begin{array}{c} 1-\frac{1}{1+{\left\{\sum_{r=1}^{4}\Phi_{r}{\left(\mu_{\sigma \left(r\right)}^{\cdot }/1-\mu_{\sigma \left(r\right)}^{\cdot }\right)}^{ℜ}\right\}}^{\left(1/ℜ\right)}},\frac{1}{1+{\left\{\sum_{r=1}^{4}\Phi_{r}{\left(1-\lambda_{\sigma \left(r\right)}^{\cdot }/\lambda_{\sigma \left(r\right)}^{\cdot }\right)}^{ℜ}\right\}}^{\left(1/ℜ\right)}},\\ \frac{-1}{1+{\left\{\sum_{r=1}^{4}\Phi_{r}{\left(1+\delta_{\sigma \left(r\right)}^{\cdot }/\left|\delta_{\sigma \left(r\right)}^{\cdot }\right|\right)}^{ℜ}\right\}}^{\left(1/ℜ\right)}} \end{array}\right)\\ =\left(\begin{array}{c} 1-\frac{1}{1+{\left\{0.2{\left(0.6145/1-0.6145\right)}^{3}+0.3{\left(0.7126/1-0.7126\right)}^{3}+0.3{\left(0.6145/1-0.6145\right)}^{3}+0.2{\left(0.1884/1-0.1884\right)}^{3}\right\}}^{\left(1/3\right)}},\\ \frac{1}{1+{\left\{0.2{\left(1-0.3855/0.3855\right)}^{3}+0.3{\left(1-0.1904/0.3179\right)}^{3}+0.3{\left(1-0.3179/0.3179\right)}^{3}+0.2{\left(1-0.3419/0.3419\right)}^{3}\right\}}^{\left(1/3\right)}},\\ \frac{-1}{1+{\left\{0.2{\left(1-0.3158/0.3158\right)}^{3}+0.3{\left(1-0.2874/0.2874\right)}^{3}+0.3{\left(1-0.2874/0.2874\right)}^{3}+0.2{\left(1-0.4180/0.4180\right)}^{3}\right\}}^{\left(1/3\right)}} \end{array}\right)\\ =\left(0.1831,0.1890,-0.2602\right). \end{array}$$

### 2.3. TF Dombi Geometric Aggregation Operators

In this section, we will propose and examine several Dombi geometric AOs, namely, the TFDWG operator and the TFDOWG operator, utilizing TFNs.

**Definition 13 .**

Let −*t*_*r*_=(*μ*_*r*_, *λ*_*r*_, *δ*_*r*_),  (*r*=1,…, *p*), be a family of TFNs. The TFDWG operator is a representation −*t*^*p*^⟶−*t* such that

(32) $$\begin{array}{c} {\text{TFDWG}}_{\Phi }\left(-t_{1},-t_{2},\ldots ,-t_{p}\right)={⊗}_{r=1}^{p}{\left(-t_{r}\right)}^{\Phi_{r}}, \end{array}$$

where Φ=(Φ_1_, Φ_2_,…,Φ_*p*_)^*T*^ is the weight vector of −*t*_*r*_,  (*r*=1,2,…, *p*) such that Φ_*r*_ > 0 and ⊕_*r*=1_^*p*^Φ_*r*_=1.

We can easily derive the following theorem from Definition 14.

**Theorem 7 .**

Let −*t*_*r*_=(*μ*_*r*_, *λ*_*r*_, *δ*_*r*_),  (*r*=1,2,…, *p*) be a collection of TFNs. Then, the aggregated value of TFNs is again a TFN, and by using TFDWG operator, we obtain

(33) $$\begin{array}{c} {\text{TFDWG}}_{\Phi }\left(-t_{1},-t_{2},\ldots ,-t_{p}\right)\\ ={⊗}_{r=1}^{p}{\left(-t_{r}\right)}^{\Phi_{r}}=\left(\begin{array}{c} \frac{1}{1+{\left\{{⊕}_{r=1}^{p}\Phi_{r}{\left(1-\mu_{r}/\mu_{r}\right)}^{ℜ}\right\}}^{\left(1/ℜ\right)}},1-\frac{1}{1+{\left\{{⊕}_{r=1}^{p}\Phi_{r}{\left(\lambda_{r}/1-\lambda_{r}\right)}^{ℜ}\right\}}^{\left(1/ℜ\right)}},\\ -1+\frac{1}{1+{\left\{{⊕}_{r=1}^{p}\Phi_{r}{\left(\left|\delta_{r}\right|/1+\delta_{r}\right)}^{ℜ}\right\}}^{\left(1/ℜ\right)}} \end{array}\right), \end{array}$$

where Φ=(Φ_1_, Φ_2_,…,Φ_*p*_)^*T*^ is the weight vector of −*t*_*r*_,  (*r*=1,2,…, *p*) such that Φ_*r*_ > 0 and ⊕_*r*=1_^*p*^Φ_*r*_=1.

**Proof**

By using mathematical induction, the proof is straightforward.

**Remark 6 .**

In Theorem 7,

(i) If *δ*_*r*_=0, for all *r*, then the (TFDWG) operator reduces to the IFDWG operator, as given below.
  (34) $$\begin{array}{c} {\text{IFDWG}}_{\Phi }\left(-t_{1},-t_{2},\ldots ,-t_{p}\right)\\ ={⊗}_{r=1}^{p}{\left(-t_{r}\right)}^{\Phi_{r}}=\left(\frac{1}{1+{\left\{{⊕}_{r=1}^{p}\Phi_{r}{\left(1-\mu_{r}/\mu_{r}\right)}^{ℜ}\right\}}^{\left(1/ℜ\right)}},1-\frac{1}{1+{\left\{{⊕}_{r=1}^{p}\Phi_{r}{\left(\lambda_{r}/1-\lambda_{r}\right)}^{ℜ}\right\}}^{\left(1/ℜ\right)}}\right). \end{array}$$
(ii) If *λ*_*r*_=0, for all *r*, then the TFDWG operator reduces to the BFDWG operator, as given below.
  (35) $$\begin{array}{c} {\text{BFDWG}}_{\Phi }\left(-t_{1},-t_{2},\ldots ,-t_{p}\right)\\ ={⊗}_{r=1}^{p}{\left(-t_{r}\right)}^{\Phi_{r}}=\left(\frac{1}{1+{\left\{{⊕}_{r=1}^{p}\Phi_{r}{\left(1-\mu_{r}/\mu_{r}\right)}^{ℜ}\right\}}^{\left(1/ℜ\right)}},-1+\frac{1}{1+{\left\{{⊕}_{r=1}^{p}\Phi_{r}{\left(\left|\delta_{r}\right|/1+\delta_{r}\right)}^{ℜ}\right\}}^{\left(1/ℜ\right)}}\right). \end{array}$$

TFDWG operators have some properties which are listed below:

P1 (idempotency property). If −*t*_*r*_=(*μ*_*r*_, *λ*_*r*_, *δ*_*r*_),  (*r*=1,…, *p*), is a family of TFNs so that they are all equal, i.e., if −*t*_*r*_=(*μ*_*r*_, *λ*_*r*_, *δ*_*r*_) = −*t*=(*μ*, *λ*, *δ*) for all *r*, then
  (36) $$\begin{array}{c} {\text{TFDWG}}_{\Phi }\left(-t_{1},-t_{2},\ldots ,-t_{r}\right)=-t. \end{array}$$
P2 (boundedness property). Let −*t*_*r*_=(*μ*_*r*_, *λ*_*r*_, *δ*_*r*_),  (*r*=1,2,3 …, *p*) be a family of TFNs and −*t*^−^=min − *t*_*r*_ and −*t*^+^=max − *t*_*r*_. Then,
  (37) $$\begin{array}{c} -t^{-}\leq {\text{TFDWG}}_{\Phi }\left(-t_{1},-t_{2},\ldots ,-t_{p}\right)\leq -t^{+}. \end{array}$$
P3 (monotonicity property). If −*t*_*r*_=(*μ*_*r*_, *λ*_*r*_, *δ*_*r*_),  (*r*=1,2,…, *p*), and −*t*_*r*_′=(*μ*_*r*_′, *λ*_*r*_′, *δ*_*r*_′),  (*r*=1,2,…, *p*), are two TFNs such that −*t*_*r*_ ≤ −*t*_*r*_′ for all *r*, then
  (38) $$\begin{array}{c} {\text{TFDWG}}_{\Phi }\left(-t_{1},-t_{2},\ldots ,-t_{p}\right)\leq {\text{TFDGW}}_{\Phi }\left(-t_{1}^{\prime },-t_{2}^{\prime },\ldots ,-t_{p}^{\prime }\right). \end{array}$$

The next section introduces the TFDOWG operator.

**Definition 14 .**

Let −*t*_*r*_=(*μ*_*r*_, *λ*_*r*_, *δ*_*r*_),  (*r*=1,2,3 …, *p*), be a family of TFNs. The TFDOWG operator is a mapping −*t*^*p*^⟶−*t* such that

(39) $$\begin{array}{c} {\text{TFDOWG}}_{w}\left(-t_{1},-t_{2},\ldots ,-t_{p}\right)={⊗}_{r=1}^{p}{\left(-t_{\sigma \left(r\right)}\right)}^{w_{r}}, \end{array}$$

where *w*=(*w*_1_, *w*_2_,…,*w*_*p*_)^*T*^ is an associated weight vector of −*t*_*r*_,  (*r*=1,2,…, *p*) such that *w*_*r*_ > 0 and ⊕_*r*=1_^*p*^*w*_*r*_=1 and (*σ*(1), *σ*(2),…, *σ*(*p*)) are the permutations of −*t*_*r*_,  (*r*=1,2,…, *p*) for which −*t*_*σ*(*r* − 1)_ ≥ −*t*_*σ*(*r*)_ for all *r*=1,2,…, *p*.

Using TFDOWG operator, we have the theorem mentioned below.

**Theorem 8 .**

Let −*t*_*r*_=(*μ*_*r*_, *λ*_*r*_, *δ*_*r*_),  (*r*=1,2,…, *p*), be a family of TFNs. The TFDOWG operator is a mapping −*t*^*p*^⟶−*t* such that

(40) $$\begin{array}{c} {\text{TFDOWG}}_{w}\left(-t_{1},-t_{2},\ldots ,-t_{p}\right)\\ ={⊗}_{r=1}^{p}{\left(-t_{\sigma \left(r\right)}\right)}^{w_{r}}=\left(\begin{array}{c} \frac{1}{1+{\left\{{⊕}_{r=1}^{p}\Phi_{r}{\left(1-\mu_{\sigma \left(r\right)}/\mu_{\sigma \left(r\right)}\right)}^{ℜ}\right\}}^{\left(1/ℜ\right)}},1-\frac{1}{1+{\left\{{⊕}_{r=1}^{p}\Phi_{r}{\left(\lambda_{\sigma \left(r\right)}/1-\lambda_{\sigma \left(r\right)}\right)}^{ℜ}\right\}}^{\left(1/ℜ\right)}},\\ -1+\frac{1}{1+{\left\{{⊕}_{r=1}^{p}\Phi_{r}{\left(\left|\delta_{\sigma \left(r\right)}\right|/1+\delta_{\sigma \left(r\right)}\right)}^{ℜ}\right\}}^{\left(1/ℜ\right)}} \end{array}\right), \end{array}$$

where *w*=(*w*_1_, *w*_2_,…,*w*_*p*_)^*T*^ is an associated weight vector of −*t*_*r*_,  (*r*=1,2,…, *p*) such that *w*_*r*_ > 0 and ⊕_*r*=1_^*p*^*w*_*r*_=1 and (*σ*(1), *σ*(2),…, *σ*(*p*)) are the permutations of −*t*_*r*_,  (*r*=1,2,…, *p*) for which −*t*_*σ*(*r* − 1)_ ≥ −*t*_*σ*(*r*)_ for all *r*=1,2,…, *p*.

**Remark 7 .**

In Theorem 8,

(i) If *δ*_*r*_=0, for all *r*, then the (TFDOWG) operator reduces to the IFDOWG operator, and
  (41) $$\begin{array}{c} {\text{IFDOWG}}_{w}\left(-t_{1},-t_{2},\ldots ,-t_{p}\right)\\ ={⊗}_{r=1}^{p}{\left(-t_{\sigma \left(r\right)}\right)}^{w_{r}}=\left(\frac{1}{1+{\left\{{⊕}_{r=1}^{p}\Phi_{r}{\left(1-\mu_{\sigma \left(r\right)}/\mu_{\sigma \left(r\right)}\right)}^{ℜ}\right\}}^{\left(1/ℜ\right)}},1-\frac{1}{1+{\left\{{⊕}_{r=1}^{p}\Phi_{r}{\left(\lambda_{\sigma \left(r\right)}/1-\lambda_{\sigma \left(r\right)}\right)}^{ℜ}\right\}}^{\left(1/ℜ\right)}}\right). \end{array}$$
(ii) If *λ*_*r*_=0, for all *r*, then the TFDOWG operator reduces to the BFDOWG operator, and
  (42) $$\begin{array}{c} {\text{BFDOWG}}_{w}\left(-t_{1},-t_{2},\ldots ,-t_{p}\right)\\ ={⊗}_{r=1}^{p}{\left(-t_{\sigma \left(r\right)}\right)}^{w_{r}}=\left(\frac{1}{1+{\left\{{⊕}_{r=1}^{p}\Phi_{r}{\left(1-\mu_{\sigma \left(r\right)}/\mu_{\sigma \left(r\right)}\right)}^{ℜ}\right\}}^{\left(1/ℜ\right)}},-1+\frac{1}{1+{\left\{{⊕}_{r=1}^{p}\Phi_{r}{\left(\left|\delta_{\sigma \left(r\right)}\right|/1+\delta_{\sigma \left(r\right)}\right)}^{ℜ}\right\}}^{\left(1/ℜ\right)}}\right). \end{array}$$

The TFDOWG operators have the following properties.

(P1) (idempotency property). If −*t*_*r*_=(*μ*_*r*_, *λ*_*r*_, *δ*_*r*_),  (*r*=1,…, *p*), is a family of TFNs such that they all equal, i.e., if −*t*_*r*_=(*μ*_*r*_, *λ*_*r*_, *δ*_*r*_) = −*t*=(*μ*, *λ*, *δ*) for all *r*, then
  (43) $$\begin{array}{c} {\text{TFDOWG}}_{\Phi }\left(-t_{1},-t_{2},\ldots ,-t_{r}\right)=-t. \end{array}$$
(P2) (boundedness property). Let −*t*_*r*_=(*μ*_*r*_, *λ*_*r*_, *δ*_*r*_), (*r*=1,2,…, *p*), be a family of TFNs and −*t*^−^=min − *t*_*r*_ and −*t*^+^=max − *t*_*r*_. Then,
  (44) $$\begin{array}{c} -t^{-}\leq {\text{TFDOWG}}_{\Phi }\left(-t_{1},-t_{2},\ldots ,-t_{p}\right)\leq -t^{+}. \end{array}$$
(P3) (monotonicity property). If −*t*_*r*_=(*μ*_*r*_, *λ*_*r*_, *δ*_*r*_), (*r*=1,2,…, *p*), and −*t*_*r*_′=(*μ*_*r*_′, *λ*_*r*_′, *δ*_*r*_′),  (*r*=1,2,…, *p*), are two TFNs such that −*t*_*r*_ ≤ −*t*_*r*_′ for all *r*, then
  (45) $$\begin{array}{c} {\text{TFDOWG}}_{\Phi }\left(-t_{1},-t_{2},\ldots ,-t_{p}\right)\leq {\text{TFDOWG}}_{\Phi }\left(-t_{1}^{\prime },-t_{2}^{\prime },\ldots ,-t_{p}^{\prime }\right). \end{array}$$

**Definition 15 .**

A TFDHWG operator of dimension *p* is a mapping TFDHWG:−*t*^*p*^⟶*t* with associated weight vector *w*=(*w*_1_, *w*_2_,…, *w*_*p*_) such that *w*_*r*_ > 0, ⊕_*r*=1_^*p*^*w*_*r*_=1, and TFDHWG operator can be evaluated as

(46) $$\begin{array}{c} {\text{TFDHWG}}_{\left(w,\Phi \right)}\left(-t_{1},-t_{2},\ldots ,-t_{p}\right)\\ ={⊗}_{r=1}^{p}{\left(-t_{\sigma \left(r\right)}^{\cdot }\right)}^{w_{r}}=\left(\begin{array}{c} \frac{1}{1+{\left\{{⊕}_{r=1}^{p}w_{r}{\left(1-\mu_{\sigma \left(r\right)}^{\cdot }/\mu_{\sigma \left(r\right)}^{\cdot }\right)}^{ℜ}\right\}}^{\left(1/ℜ\right)}},1-\frac{1}{1+{\left\{{⊕}_{r=1}^{p}w_{r}{\left(\lambda_{\sigma \left(r\right)}^{\cdot }/1-\lambda_{\sigma \left(r\right)}^{\cdot }\right)}^{ℜ}\right\}}^{\left(1/ℜ\right)}},\\ -1+\frac{1}{1+{\left\{{⊕}_{r=1}^{p}w_{r}{\left(\left|\delta_{\sigma \left(r\right)}^{\cdot }\right|/1-\delta_{\sigma \left(r\right)}^{\cdot }\right)}^{ℜ}\right\}}^{\left(1/ℜ\right)}} \end{array}\right), \end{array}$$

where −*t*_*σ*(*r*)_^·^ is the *r*^th^ largest weighted tripolar fuzzy number, denoted by −*t*_*r*_^·^, and (−*t*_*r*_^·^=*p*Φ − *t*_*r*_,  *r*=1,2,…, *p*) and Φ=(Φ_1_, Φ_2_,…,Φ_*p*_)^*T*^ are the weight vectors of −*t*_*r*_^·^ with Φ_*r*_ > 0, ⊕_*r*=1_^*p*^Φ_*r*_=1, where *p* is the balancing coefficient. A TFDHWG operator has some special cases:

- When *w*=((1/*p*), (1/*p*),…, (1/*p*)), then (TFDWG) operator is a special case of TFDHWG operator.
- When Φ=((1/*p*), (1/*p*),…, (1/*p*)), then (TFDOWG) operator becomes a special case of TFDHWG operator.

As a result, the TFDHG operator is a generalization of both the TFDWG and TFDOWG operators, reflecting the degrees of the provided arguments as well as their ordered locations.

**Remark 8 .**

In Definition 15,

(i) If *δ*_*r*_=0, for all *r*=1,2,…, *p*, then TFDHWG operator reduces to IFDHWG operator and
  (47) $$\begin{array}{c} {\text{IFDHWG}}_{\left(w,\Phi \right)}\left(-t_{1},-t_{2},\ldots ,-t_{p}\right)\\ ={⊗}_{r=1}^{p}{\left(-t_{\sigma \left(r\right)}^{\cdot }\right)}^{w_{r}}=\left(\frac{1}{1+{\left\{{⊕}_{r=1}^{p}w_{r}{\left(1-\mu_{\sigma \left(r\right)}^{\cdot }/\mu_{\sigma \left(r\right)}^{\cdot }\right)}^{ℜ}\right\}}^{\left(1/ℜ\right)}},1-\frac{1}{1+{\left\{{⊕}_{r=1}^{p}w_{r}{\left(\lambda_{\sigma \left(r\right)}^{\cdot }/1-\lambda_{\sigma \left(r\right)}^{\cdot }\right)}^{ℜ}\right\}}^{\left(1/ℜ\right)}}\right). \end{array}$$
(ii) If *λ*_*r*_=0, for all *r*, then TFDHWG operator reduces to BFDHWG operator and
  (48) $$\begin{array}{c} {\text{BFDHWG}}_{\left(w,\Phi \right)}\left(-t_{1},-t_{2},\ldots ,-t_{p}\right)\\ ={⊗}_{r=1}^{p}{\left(-t_{\sigma \left(r\right)}^{\cdot }\right)}^{w_{r}}=\left(\frac{1}{1+{\left\{{⊕}_{r=1}^{p}w_{r}{\left(1-\mu_{\sigma \left(r\right)}^{\cdot }/\mu_{\sigma \left(r\right)}^{\cdot }\right)}^{ℜ}\right\}}^{\left(1/ℜ\right)}},-1+\frac{1}{1+{\left\{{⊕}_{r=1}^{p}w_{r}{\left(\left|\delta_{\sigma \left(r\right)}^{\cdot }\right|/1-\delta_{\sigma \left(r\right)}^{\cdot }\right)}^{ℜ}\right\}}^{\left(1/ℜ\right)}}\right). \end{array}$$

For the validity of Definition 15, we consider the following example.

**Example 2 .**

Let −*t*_1_=(0.5, 0.4, −0.3), −*t*_2_=(0.6, 0.3, −0.3), −*t*_3_=(0.7, 0.2, −0.3), and −*t*_4_=(0.2, 0.3, −0.4) be four TFNs and Φ=(0.20, 0.30, 0.30, 0.20)^*T*^ and *w*=(0.2, 0.1, 0.3, 0.4)^*T*^ be the weight vector of TFNs and associated weight vector, respectively. Then, by Definition 15, for aggregated value of TFNs for (*ℜ*=3) and by using TFDHG operator, we have

(49) $$\begin{array}{c} -t_{1}^{\cdot }=\left(\begin{array}{c} \frac{1}{1+{\left\{4\times 0.2{\left(1-0.5/0.5\right)}^{3}\right\}}^{\left(1/3\right)}},1-\frac{1}{1+{\left\{4\times 0.2{\left(0.4/1-0.4\right)}^{3}\right\}}^{\left(1/3\right)}},\\ -1+\frac{1}{1+{\left\{4\times 0.20{\left(0.3/1-0.3\right)}^{3}\right\}}^{\left(1/3\right)}} \end{array}\right)\\ =\left(0.4814,0.4179,-0.3158\right),\\ -t_{2}^{\cdot }=\left(\begin{array}{c} \frac{1}{1+{\left\{4\times 0.3{\left(1-0.6/0.6\right)}^{3}\right\}}^{\left(1/3\right)}},1-\frac{1}{1+{\left\{4\times 0.3{\left(0.3/1-0.3\right)}^{3}\right\}}^{\left(1/3\right)}},\\ -1+\frac{1}{1+{\left\{4\times 0.30{\left(0.3/1-0.3\right)}^{3}\right\}}^{\left(1/3\right)}} \end{array}\right)\\ =\left(0.5820,0.3158,-0.3158\right),\\ -t_{3}^{\cdot }=\left(\begin{array}{c} \frac{1}{1+{\left\{4\times 0.3{\left(1-0.7/0.7\right)}^{3}\right\}}^{\left(1/3\right)}},1-\frac{1}{1+{\left\{4\times 0.3{\left(0.2/1-0.2\right)}^{3}\right\}}^{\left(1/3\right)}},\\ -1+\frac{1}{1+{\left\{4\times 0.30{\left(0.3/1-0.3\right)}^{3}\right\}}^{\left(1/3\right)}} \end{array}\right)\\ =\left(0.6841,0.2121,-0.3158\right),\\ -t_{4}^{\cdot }=\left(\begin{array}{c} \frac{1}{1+{\left\{4\times 0.2{\left(1-0.2/0.2\right)}^{3}\right\}}^{\left(1/3\right)}},1-\frac{1}{1+{\left\{4\times 0.2{\left(0.3/1-0.3\right)}^{3}\right\}}^{\left(1/3\right)}},\\ -1+\frac{1}{1+{\left\{4\times 0.20{\left(0.4/1-0.4\right)}^{3}\right\}}^{\left(1/3\right)}} \end{array}\right)\\ =\left(0.1883,0.3158,-0.4179\right). \end{array}$$

Scores of −*t*_*r*_^·^,  (*r*=1,2,3,4) can be approximated:

(50) $$\begin{array}{c} Ⓢ\left(-t_{1}^{\prime }\right)=\frac{1+0.4814+0.4179-0.3158}{3}=0.5278,\\ Ⓢ\left(-t_{2}^{\prime }\right)=\frac{1+0.5820+0.3158-0.3158}{3}=0.5273,\\ Ⓢ\left(-t_{3}^{\prime }\right)=\frac{1+0.6841+0.2121-0.3158}{3}=0.5268,\\ Ⓢ\left(-t_{4}^{\prime }\right)=\frac{1+0.1883+0.3851-0.4179}{3}=0.3620. \end{array}$$

Since Ⓢ(−*t*_1_^·^) > Ⓢ(−*t*_2_^·^) > Ⓢ(−*t*_3_^·^) > Ⓢ(−*t*_4_^·^), then we have

(51) $$\begin{array}{c} -t_{\sigma \left(1\right)}^{\cdot }=-t_{1}^{\cdot }=\left(0.4814,0.4179,-0.3158\right),-t_{\sigma \left(2\right)}^{\cdot }=-t_{2}^{\cdot }=\left(0.5820,0.3158,-0.3158\right),\\ -t_{\sigma \left(3\right)}^{\cdot }=-t_{3}^{\cdot }=\left(0.6841,0.2121,-0.3150\right),-t_{\sigma \left(4\right)}^{\cdot }=-t_{4}^{\cdot }=\left(0.1883,0.3158,-0.4179\right). \end{array}$$

According to Definition 15, the aggregated values under TFDHWG operators for (*R*=3) are calculated as

(52) $$\begin{array}{c} {\text{TFDHWG}}_{\left(w,\Phi \right)}\left(-t_{1},-t_{2},\ldots ,-t_{4}\right)\\ ={⊗}_{r=1}^{4}{\left(-t_{\sigma \left(r\right)}^{\cdot }\right)}^{w_{r}}=\left(\begin{array}{c} \frac{1}{1+{\left\{\sum_{r=1}^{4}w_{r}{\left(1-\mu_{\sigma \left(r\right)}^{\cdot }/\mu_{\sigma \left(r\right)}^{\cdot }\right)}^{3}\right\}}^{\left(1/3\right)}},1-\frac{1}{1+{\left\{\sum_{r=1}^{4}{\left(\lambda_{\sigma \left(r\right)}^{\cdot }/1-\lambda_{\sigma \left(r\right)}^{\cdot }\right)}^{3}\right\}}^{\left(1/3\right)}},\\ -1+\frac{1}{1+{\left\{\sum_{r=1}^{4}{\left(\left|\delta_{\sigma \left(r\right)}^{\cdot }\right|/1+\delta_{\sigma \left(r\right)}^{\cdot }\right)}^{3}\right\}}^{\left(1/3\right)}} \end{array}\right)\\ =\left(\begin{array}{c} \frac{1}{1+{\left\{0.2{\left(1-0.4814/0.4814\right)}^{3}+0.1{\left(1-0.5820/0.5820\right)}^{3}+0.3{\left(1-0.6841/0.6841\right)}^{3}+0.4{\left(1-0.1883/0.1883\right)}^{3}\right\}}^{\left(1/3\right)}},\\ 1-\frac{1}{1+{\left\{0.2{\left(0.4179/1-0.4179\right)}^{3}+0.1{\left(0.3158/1-0.3158\right)}^{3}+0.3{\left(0.2121/1-0.2121\right)}^{3}+0.4{\left(0.3158/1-0.3158\right)}^{3}\right\}}^{\left(1/3\right)}},\\ -1+\frac{1}{1+{\left\{0.2{\left(0.3158/1-0.3158\right)}^{3}+0.1{\left(0.3158/1-0.3158\right)}^{3}+0.3{\left(0.3158/1-0.3158\right)}^{3}+0.4{\left(0.4179/1-0.4179\right)}^{3}\right\}}^{\left(1/3\right)}} \end{array}\right)\\ =\left(0.0799,0.2351,-0.3452\right). \end{array}$$

## 3. Models for MADM with TF Information

To solve a MADM problem using TF information, we will use the TFDA operators established in the preceding sections. The MADM problem is represented using the following technique or notations for prospective evaluation of developing technology commercialization using TF information. Let *A*={*A*_1_, *A*_2_,…, *A*_*m*_} present a discrete set of alternatives and *G*={*G*_1_, *G*_2_,…, *G*_*n*_}, the set of attributes. Let Φ=(Φ_1_, Φ_2_,…, Φ_*n*_) be the weight of attributes in the form of real numbers with the conditions Φ_*j*_ > 0 and ∑_*j*=1_^*n*^Φ_*j*_=1. Suppose that $M={\left({\tilde{m}}_{ij}\right)}_{m\times n}={\left(\mu_{ij},\lambda_{ij},\delta_{ij}\right)}_{m\times n}$ is the TF decision matrix, where *μ*_*ij*_ represent the degree of membership, *λ*_*ij*_ represent the degree of non-membership, and *δ*_*ij*_ denote the degree of negative membership such that, *μ*_*ij*_+*λ*_*ij*_ ≤ 1 and *μ*_*ij*_, *λ*_*ij*_ ⊂ [0,1] and *δ*_*ij*_ ⊂ [−1,0], (*i*=1,2,…, *n*) and (*j*=1,2,…, *m*). The process of utilizing the TFDWA (or TFDWG) operator to solve an MADM problem is listed below (Algorithm 1).

## 4. Illustrative Example

To present the practical output of the constructed model, we consider the MADM problem (adapted from [27]) of the ERP systems. We suppose that an organization wants to employ the ERP systems. The first step for the ERP system is to construct a team of experts which contained CIO and two other senior experts from the source institute. The expert's team collects all the data regarding ERP vendors and system, in the form of TFS. Secondly, the team selects five potential ERP systems, treated as *A*_*i*_,  (*i*=1,2,3,4,5), as candidates. The team also imposes four attributes for the evaluation of this MADM problem of *A*_*i*_ (*i*=1,2,3,4,5):

- *G*_1_ = function and technology.
- *G*_2_ = strategic fitness.
- *G*_3_ = vendor's reputation.
- *G*_4_ = vendor's ability.

The expert team gave some weighting for the selection of optimal candidate as Φ=(0.2, 0.1, 0.3, 0.4), and the information collected is in the form of TFSs, satisfying the above four attributes. The rating of the team is presented in the matrix given below.

To find the most favorable ERP systems, we employ the TFDWA operator (or TFDWG operator) in the following to construct a solution to MADM problems based on TF information, which may be summarized as follows.

*Step 1*. Let *ℜ*=1. By applying the TFDWA operator, we compute the overall preference values ${\tilde{m}}_{i}$ of the ERP system *A*_*i*_ (*i*=1,2,3,4,5):
  (53) $$\begin{array}{c} {\tilde{m}}_{1}=\left(0.0013,0.9455,-0.9871\right),\\ {\tilde{m}}_{2}=\left(0.0010,0.9800,-0.9964\right),\\ {\tilde{m}}_{3}=\left(0.0004,0.9788,-0.8852\right),\\ {\tilde{m}}_{4}=\left(0.0001,0.9976,-0.9936\right),\\ {\tilde{m}}_{5}=\left(0.0037,0.9562,-0.9814\right). \end{array}$$
*Step 2*. Find the score values $Ⓢ\left({\tilde{m}}_{i}\right),\;\left(i=1,2,3,4,5\right)$, of the overall TF numbers, TFNs, ${\tilde{m}}_{i},\;\left(i=1,2,3,4,5\right)$:
  (54) $$\begin{array}{c} Ⓢ\left({\tilde{m}}_{1}\right)=0.3199,\\ Ⓢ\left({\tilde{m}}_{2}\right)=0.3282,\\ Ⓢ\left({\tilde{m}}_{3}\right)=0.3646,\\ Ⓢ\left({\tilde{m}}_{4}\right)=0.3347,\\ Ⓢ\left({\tilde{m}}_{5}\right)=0.3261. \end{array}$$
*Step 3*. Rank all the ERP systems *A*_*i*_,  (*i*=1,2,3,4,5), according to the respective score values of the overall tripolar fuzzy numbers, and we get *A*_3_ > *A*_4_ > *A*_2_ > *A*_5_ > *A*_1_.
*Step 4*. According to score values, *A*_3_ is the most considerable ERP system.

If we use the TFDWG operator instead of TFDWA operator, then we solve the problem similarly as above:

*Step 1*. For *ℜ*=1, aggregate all TFNs via the TFDWG operator to derive the overall TFNs ${\tilde{m}}_{i}\;\left(i=1,2,3,4,5\right)$ of the ERP system:
  (55) $$\begin{array}{c} {\tilde{m}}_{1}=\left(0.9959,0.0000,-0.0004\right),\\ {\tilde{m}}_{2}=\left(0.9944,0.0002,-0.0015\right),\\ {\tilde{m}}_{3}=\left(0.9875,0.0002,-0.0000\right),\\ {\tilde{m}}_{4}=\left(0.9674,0.0023,-0.0008\right),\\ {\tilde{m}}_{5}=\left(0.9984,0.0001,-0.0003\right). \end{array}$$
*Step 2*. Calculate the score values $Ⓢ\left({\tilde{m}}_{i}\right),\;\left(i=1,2,3,4,5\right)$, of the overall TF numbers, TFNs, ${\tilde{m}}_{i},\;\left(i=1,2,3,4,5\right)$:
  (56) $$\begin{array}{c} Ⓢ\left({\tilde{m}}_{1}\right)=0.6651,\\ Ⓢ\left({\tilde{m}}_{2}\right)=0.6643,\\ Ⓢ\left({\tilde{m}}_{3}\right)=0.6625,\\ Ⓢ\left({\tilde{m}}_{4}\right)=0.6563,\\ Ⓢ\left({\tilde{m}}_{5}\right)=0.6660. \end{array}$$
*Step 3*. Rank all the ERP systems *A*_*i*_,  (*i*=1,2,3,4,5), according to the respective score values of the overall TF numbers, and we get Ⓢ*A*_5_ > Ⓢ*A*_1_ > Ⓢ*A*_2_ > Ⓢ*A*_3_ > Ⓢ*A*_4_.
*Step 4*. By the score values, *A*_5_ is the most ideal ERP system.

Based on the above discussion, it is determined that, while ranking values of the alternatives change when utilizing the TFDWA (TFDWG) operator, the ranking orders of the ERP system did not remain the same, i.e., the most ideal ERP system through using TFDWA operator is *A*_4_, while using TFDWG operator, it is *A*_5_. The reason for different optimal alternatives is the use of different methods in the decision process.

In Figure 1, the comparison of the ERP system is shown, where it is observed that the graph of TFDWA operator (green line) has some fluctuations in the middle values of ranking order of ERP system while the graph of TFDWG operator (brown line) is stable. This means that the ranking order of ERP systems is more stable in TFDWG operator as compared to the ranking order of ERP systems in TFDWA operator.

### 4.1. Influence of Parameter

To describe the impact of the operational parameters *ℜ* on MADM outcomes, we will rank the alternatives using different values of *ℜ*. The results of score function and ranking order of the ERP system *A*_*i*_(*i*=1,2,3,4,5) in the range of *ℜ* ∈ [1,10] applying TFDWA and TFDWG operators are presented. The corresponding scores and ranking of the ERP system *A*_*i*_,  (*i*=1,2,3,4,5), are shown in Tables 1 and 2.

Table 3 shows that altering the value of *ℜ* in the TFDWA operator changes the ranking orders, and the associated best alternatives are not similar. Several ranking orders of the alternatives for subintervals of [2, 30] by using TFDWA and TFDWG operators of the operational parameter *ℜ* are shown in Tables 2 and 4.

Ranking orders of the alternatives for subintervals of [2, 30] by using TFDWG operators of the operational parameter *ℜ* are shown in Table 5.

The corresponding graphs in Figures 2 and 3 are provided to diagnose the influence of parameter *ℜ*  ∈  [1, 10] on the ranking of alternatives in TFDWA and TFDWG operators.

From Figures 2 and 3, we observe that the ranking order of the ERP systems in TFDWA operator (Figure 2) has more fluctuations than the ranking order of alternatives in TFDWG operators (Figure 3). Therefore, the proposed method of TFDWG operator produced stable results of the ERP system.

### 4.2. Comparative Analysis

To compare the developed models with the existing literature to describe the advantages of the proposed models, we consider the following two special cases of the suggested models, given in Examples 1 and 2. In Example 1, we dropped the implicit counter property from the information given in Table 1 and the reduced matrix becomes the IF information which is given in Table 6.

**Example 3 .**

Recall the TF information decision matrix given in Table 1. The modified decision matrix contained IF information given in Table 6, and the normalized decision matrix is shown in Table 7, respectively.

By applying IFDWA and IFDWG operators on Table 7, the aggregated IFNs are summarized in Table 8.

By calculating the score values of the aggregated IFNs of Table 9, we get the following table.

In Table 10, a comparison of the ranking of alternatives by using IFDWA operator and TFDWA operator is shown, and the graphical view of these operators is highlighted in Figure 4.

From Figure 4, we can see that the ranking order of alternatives for the TFDWA operator (brown line) is stable from *A*_1_ to *A*_2_, increasing from *A*_2_ to *A*_3_, decreasing from *A*_3_ to *A*_4_, and stable from *A*_4_ to *A*_5_. From *A*_4_ it becomes stable. On the other hand, if we consider the IFDWA operator (green line), the ranking order of alternatives is decreasing continuously from *A*_1_ to *A*_4_ and increasing from *A*_4_ to *A*_5_, and hence we observe no stability in ranking produced by IFDWA operator. Therefore, the proposed method of TFDWA operator gives more stable ranking than the existing methods in literature.

A comparison of the ranking of alternatives by using IFDWG operator and TFDWG operator is shown in Table 11, and the graphical view of these operators is highlighted in Figure 5.

From Figure 5, it is clearly seen that the ranking of alternatives in IFDWG operator (green line) is stable from *A*_1_ to *A*_5_. Similarly, the ranking in TFDWG operator (brown line) is stable from *A*_1_ to *A*_5_. Therefore, the stability of our proposed operator is similar to the stability of existing IFDWG operator, but the proposed TFDWG operator is more advanced than the existing operator, as it is a generalization of both the notions of IFNs and BFNs and can handle problems involving IFN and BFN in the single model.

Now, we discuss the case of proposed operators by dropping the degree of non-membership from the information given in the decision matrix of Table 1. The following example illustrate the case of dropping the degree of non-membership.

**Example 4 .**

Reconsider the decision matrix given in Table 1 and drop the non-membership degree from each triplet of this matrix. The modified matrix is reduced to a BF decision matrix given in Table 12.

For the comparison of the proposed models, we apply BFDWA and BFDWG operators on Table 12 and the aggregated BFNs are summarized in Table 13.

The score values of the aggregated BFNs are summarized in Table 14.

The ranking of alternatives by using BFDWA/BFDWG operator is shown in Table 15.

In Table 16, we compare the ranking order of alternatives obtained by the proposed method and BFDWA/BFDWG operators.

In Figures 6 and 7, we compared the proposed operators and existing operators of BFDWA/BFDWG operators.

From Figure 7, it is clearly seen that the ranking of alternatives using BFDWA operator (brown line) and TFDWA operator (green line) is not fully stable in between *A*_1_ to *A*_5_.

From Figure 7, we observed that the ranking order of alternatives in BFDWG operator (green line) and TFDWG operator (brown line) is stable. This means that the proposed operators and existing operator behave similar. But the proposed operators are generalization of both the IFS and BFS, which combine both the notions into a single model.

## 5. Conclusion

In this article, we addressed MADM problems with TF information. From the inspiration of Dombi operations, we incorporated arithmetic and geometric operations to develop certain TF Dombi aggregation operators:

- TFDWA operator.
- TFDOWA operator.
- TFDHWA operator.
- PFDWG operator.
- TFDOWG operator.
- TFDHWG operator.

Different aspects of these suggested operators are highlighted. Then, we utilized these operators to broaden a few mechanisms to cope with MADM problems. Ultimately, a realistic example of an ERP system is provided to develop the strategy and show the effectiveness of the proposed method. In future research, we will investigate DM theory, risk theory, and other areas in an ambiguous environment for the suggested tripolarity models.

The method introduced in this paper is a generalization of IF and BF environments, and the present model deals with the tripolar fuzzy environment. The existing methods of IF sets and BF sets [5, 30] for MADM problems have restrictions; in IFS, we cannot discuss the implicit counter property of objects while the BFS models failed to consider the non-membership property of objects in decision process, and definitely these deficiencies in IF models as well as in BF models will lose the information in the process. The present method combines the two concepts of IF and BF models together. In a nutshell, the suggested MADM technique for TFDWA and TFDWGA operators has improved DM reliability. Our suggested approaches are more comprehensive and adaptable than conventional methods for controlling IF and BF models. We compared our method with Dombi's method [30] and Xu and Yager's method [5]. The comparative results are shown in Table 17. As a conclusion, our suggested approaches are more flexible and adaptable than available methods for controlling IF and BF MADM challenges.

## Figures and Tables

**Figure 1:** Graphs of TFDWA and TFDWG operators.

**Figure 2:** Graphs of alternatives in TFDWA operator (<2 [2, 30]).

**Figure 3:** Graphs of alternatives in TFDWG operator (<2 [2, 30]).

**Figure 4:** Comparison of ranking order in TFDWA and IFDWA operators.

**Figure 5:** Ranking order of alternatives in TFDWG and IFDWG operators.

**Figure 6:** Comparison of alternatives in TFDWA and BFDWA operators.

**Figure 7:** Comparison of alternatives in BFDWG and TFDWG operators.

**Algorithm 1:** MADM steps.

**Table 1:** Tripolar fuzzy (TF) decision matrix with its values.

TF matrix values
$M=\left[\begin{array}{cccc} \left(0.7,0.2,-0.3\right) & \left(0.2,0.4,-0.8\right) & \left(0.2,0.5,-0.3\right) & \left(0.8,0.2,-0.2\right)\\ \left(0.6,0.3,-0.4\right) & \left(0.3,0.6,-0.5\right) & \left(0.5,0.3,-0.4\right) & \left(0.4,0.3,-0.6\right)\\ \left(0.4,0.5,-0.2\right) & \left(0.4,0.4,-0.1\right) & \left(0.3,0.2,-0.5\right) & \left(0.5,0.4,-0.4\right)\\ \left(0.2,0.6,-0.6\right) & \left(0.3,0.4,-0.7\right) & \left(0.4,0.6,-0.2\right) & \left(0.5,0.4,-0.3\right)\\ \left(0.7,0.3,-0.3\right) & \left(0.5,0.4,-0.4\right) & \left(0.5,0.3,-0.4\right) & \left(0.4,0.3,-0.4\right) \end{array}\right]$

**Table 2:** Ranking order in TFDWA operator.

*ℜ*	Ranking orders
*ℜ* ∈ 1,2]	Ⓢ*A*_3_ > Ⓢ*A*_4_ > Ⓢ*A*_2_ > Ⓢ*A*_5_ > Ⓢ*A*_1_
*ℜ* ∈ (2,4]	Ⓢ*A*_3_ > Ⓢ*A*_4_ > Ⓢ*A*_1_ > Ⓢ*A*_5_ > Ⓢ*A*_2_
*ℜ* ∈ (4,5]	Ⓢ*A*_5_ > Ⓢ*A*_3_ > Ⓢ*A*_4_ > Ⓢ*A*_1_ > Ⓢ*A*_2_
*ℜ* ∈ (5,6]	Ⓢ*A*_4_ > Ⓢ*A*_3_ > Ⓢ*A*_5_ > Ⓢ*A*_1_ > Ⓢ*A*_2_
*ℜ* ∈ (6,10]	Ⓢ*A*_5_ > Ⓢ*A*_4_ > Ⓢ*A*_3_ > Ⓢ*A*_1_ > Ⓢ*A*_2_

**Table 3:** The ERP's ranking order for various working parameters in TFDWA operator.

*ℜ*	Ⓢ $\left({\tilde{m}}_{1}\right)$, Ⓢ $\left({\tilde{m}}_{2}\right)$, Ⓢ $\left({\tilde{m}}_{3}\right)$, Ⓢ $\left({\tilde{m}}_{4}\right)$, Ⓢ $\left({\tilde{m}}_{5}\right)$	Ranking order
1	0.3199,0.3282,0.3646,0.3347,0.3261	Ⓢ*A*_3_ > Ⓢ*A*_4_ > Ⓢ*A*_2_ > Ⓢ*A*_5_ > Ⓢ*A*_1_
2	0.2326,0.2652,0.4763,0.3574,0.2887	Ⓢ*A*_3_ > Ⓢ*A*_4_ > Ⓢ*A*_5_ > Ⓢ*A*_2_ > Ⓢ*A*_1_
3	0.2438,0.2300,0.4522,0.3848,0.2335	Ⓢ*A*_3_ > Ⓢ*A*_4_ > Ⓢ*A*_1_ > Ⓢ*A*_5_ > Ⓢ*A*_2_
4	0.2730,0.2279,0.4324,0.4018,0.2091	Ⓢ*A*_3_ > Ⓢ*A*_4_ > Ⓢ*A*_1_ > Ⓢ*A*_5_ > Ⓢ*A*_2_
5	0.2968,0.2354,0.4221,0.4114,0.4257	Ⓢ*A*_5_ > Ⓢ*A*_3_ > Ⓢ*A*_4_ > Ⓢ*A*_1_ > Ⓢ*A*_2_
6	0.3146,0.2446,0.4166,0.4171,0.3896	Ⓢ*A*_4_ > Ⓢ*A*_3_ > Ⓢ*A*_5_ > Ⓢ*A*_1_ > Ⓢ*A*_2_
7	0.3281,0.2531,0.4135,0.4206,0.4253	Ⓢ*A*_5_ > Ⓢ*A*_4_ > Ⓢ*A*_3_ > Ⓢ*A*_1_ > Ⓢ*A*_2_
8	0.3386,0.2607,0.4118,0.4230,0.4367	Ⓢ*A*_5_ > Ⓢ*A*_4_ > Ⓢ*A*_3_ > Ⓢ*A*_1_ > Ⓢ*A*_2_
9	0.3470,0.2671,0.4107,0.4246,0.4457	Ⓢ*A*_5_ > Ⓢ*A*_4_ > Ⓢ*A*_3_ > Ⓢ*A*_1_ > Ⓢ*A*_2_
10	0.3537,0.2727,0.4101,0.4257,0.4529	Ⓢ*A*_5_ > Ⓢ*A*_4_ > Ⓢ*A*_3_ > Ⓢ*A*_1_ > Ⓢ*A*_2_

**Table 4:** Ranking order in TFDWG operator.

*ℜ*	Ranking order
*ℜ* ∈ 0,3]	Ⓢ*A*_5_ > Ⓢ*A*_1_ > Ⓢ*A*_2_ > Ⓢ*A*_3_ > Ⓢ*A*_4_
*ℜ* ∈ (3,5]	Ⓢ*A*_3_ > Ⓢ*A*_4_ > Ⓢ*A*_1_ > Ⓢ*A*_5_ > Ⓢ*A*_2_
*ℜ* ∈ (5,7]	Ⓢ*A*_5_ > Ⓢ*A*_1_ > Ⓢ*A*_2_ > Ⓢ*A*_3_ > Ⓢ*A*_4_
*ℜ* ∈ (7,8]	Ⓢ*A*_5_ > Ⓢ*A*_1_ > Ⓢ*A*_3_ > Ⓢ*A*_4_ > Ⓢ*A*_2_
*ℜ* ∈ (8,10]	Ⓢ*A*_5_ > Ⓢ*A*_1_ > Ⓢ*A*_3_ > Ⓢ*A*_4_ > Ⓢ*A*_2_

**Table 5:** Ranking order for various working parameters in TFDWG operator.

*ℜ*	Ⓢ $\left({\tilde{m}}_{1}\right)$, Ⓢ $\left({\tilde{m}}_{2}\right)$, Ⓢ $\left({\tilde{m}}_{3}\right)$, Ⓢ $\left({\tilde{m}}_{4}\right)$, Ⓢ $\left({\tilde{m}}_{5}\right)$	Ranking order
1	0.6651,0.6643,0.6625,0.6563,0.6660	Ⓢ*A*_5_ > Ⓢ*A*_1_ > Ⓢ*A*_2_ > Ⓢ*A*_3_ > Ⓢ*A*_4_
2	0.6385,0.6238,0.5998,0.5406,0.6552	Ⓢ*A*_5_ > Ⓢ*A*_1_ > Ⓢ*A*_2_ > Ⓢ*A*_3_ > Ⓢ*A*_4_
3	0.5982,0.5651,0.5331,0.4726,0.6369	Ⓢ*A*_5_ > Ⓢ*A*_1_ > Ⓢ*A*_2_ > Ⓢ*A*_3_ > Ⓢ*A*_4_
4	0.5650,0.5187,0.4941,0.4495,0.6198	Ⓢ*A*_3_ > Ⓢ*A*_4_ > Ⓢ*A*_1_ > Ⓢ*A*_5_ > Ⓢ*A*_2_
5	0.5403,0.4855,0.4718,0.4495,0.6195	Ⓢ*A*_3_ > Ⓢ*A*_4_ > Ⓢ*A*_1_ > Ⓢ*A*_5_ > Ⓢ*A*_2_
6	0.5222,0.4615,0.4492,0.4349,0.5857	Ⓢ*A*_5_ > Ⓢ*A*_1_ > Ⓢ*A*_2_ > Ⓢ*A*_3_ > Ⓢ*A*_4_
7	0.5083,0.4438,0.4492,0.4349,0.5857	Ⓢ*A*_5_ > Ⓢ*A*_1_ > Ⓢ*A*_2_ > Ⓢ*A*_3_ > Ⓢ*A*_4_
8	0.4977,0.4302,0.4430,0.4360,0.5784	Ⓢ*A*_5_ > Ⓢ*A*_1_ > Ⓢ*A*_3_ > Ⓢ*A*_4_ > Ⓢ*A*_2_
9	0.4892,0.4194,0.4385,0.4333,0.5725	Ⓢ*A*_5_ > Ⓢ*A*_1_ > Ⓢ*A*_3_ > Ⓢ*A*_4_ > Ⓢ*A*_2_
10	0.4823,0.4108,0.4351,0.4329,0.5676	Ⓢ*A*_5_ > Ⓢ*A*_1_ > Ⓢ*A*_3_ > Ⓢ*A*_4_ > Ⓢ*A*_2_

**Table 6:** Intuitionistic fuzzy (IF) decision matrix.

IF matrix values
$M^{\prime }=\left[\begin{array}{cccc} \left(\text{0.}7\text{,0.}2\right) & \left(\text{0.}2\text{,0.}4\right) & \left(\text{0.}2\text{,0.}5\right) & \left(\text{0.}8\text{,0.}2\right)\\ \left(\text{0.}6\text{,0.}3\right) & \left(\text{0.}3\text{,0.}6\right) & \left(\text{0.}5\text{,0.}3\right) & \left(\text{0.}4\text{,0.}3\right)\\ \left(\text{0.}4\text{,0.}5\right) & \left(\text{0.}4\text{,0.}4\right) & \left(\text{0.}3\text{,0.}2\right) & \left(\text{0.}5\text{,0.}4\right)\\ \left(\text{0.}2\text{,0.}6\right) & \left(\text{0.}3\text{,0.}4\right) & \left(\text{0.}4\text{,0.}6\right) & \left(\text{0.}5\text{,0.}4\right)\\ \left(\text{0.}7\text{,0.}3\right) & \left(\text{0.}5\text{,0.}4\right) & \left(\text{0.}5\text{,0.}3\right) & \left(\text{0.}4\text{,0.}3\right) \end{array}\right]$

**Table 7:** Normalized intuitionistic fuzzy (NIF) decision matrix.

NIF matrix values
$M=\left[\begin{array}{cccc} \left(\text{0.}7\text{,0.}2\right) & \left(\text{0.}4\text{,0.}2\right) & \left(\text{0.}2\text{,0.}5\right) & \left(\text{0.}8\text{,0.}2\right)\\ \left(\text{0.}6\text{,0.}3\right) & \left(\text{0.}6\text{,0.}3\right) & \left(\text{0.}5\text{,0.}3\right) & \left(\text{0.}4\text{,0.}3\right)\\ \left(\text{0.}4\text{,0.}5\right) & \left(\text{0.}4\text{,0.}4\right) & \left(\text{0.}3\text{,0.}2\right) & \left(\text{0.}5\text{,0.}4\right)\\ \left(\text{0.}2\text{,0.}6\right) & \left(\text{0.}4\text{,0.}3\right) & \left(\text{0.}4\text{,0.}6\right) & \left(\text{0.}5\text{,0.}4\right)\\ \left(\text{0.}7\text{,0.}3\right) & \left(\text{0.}4\text{,0.}5\right) & \left(\text{0.}5\text{,0.}3\right) & \left(\text{0.}4\text{,0.}3\right) \end{array}\right]$

**Table 8:** Aggregated IFNs using IFDWA and IFDWG operators.

Alternatives	BFDWA operator	BFDWG operator
*A*_1_	(0.0037, 0.8668)	(0.9984, 0.0000)
*A*_2_	(0.0030, 0.9335)	(0.9964, 0.0000)
*A*_3_	(0.0004, 0.9788)	(0.9875, 0.0002)
*A*_4_	(0.0002, 0.9962)	(0.9788, 0.0015)
*A*_5_	(0.0024, 0.9704)	(0.9976, 0.0001)

**Table 9:** Score values of IFNs using IFDWA and IFDWG operators.

Alternatives	IFDWA operator	IFDWG operator
*A*_1_	0.0684	0.9992
*A*_2_	0.0347	0.9982
*A*_3_	0.0108	0.9936
*A*_4_	0.0020	0.9886
*A*_5_	0.0160	0.9987

*Ranking order of alternatives*		
IFDWA operator	Ⓢ*A*_1_ > Ⓢ*A*_2_ > Ⓢ*A*_5_ > Ⓢ*A*_3_ > Ⓢ*A*_4_	
IFDWG operator	Ⓢ*A*_1_ > Ⓢ*A*_5_ > Ⓢ*A*_2_ > Ⓢ*A*_3_ > Ⓢ*A*_4_	

**Table 10:** Ranking of alternatives using IFDWA and TFDWA operators.

IFDWA operator	Ⓢ*A*_1_ > Ⓢ*A*_2_ > Ⓢ*A*_5_ > Ⓢ*A*_3_ > Ⓢ*A*_4_
TFDWA operator	Ⓢ*A*_3_ > Ⓢ*A*_4_ > Ⓢ*A*_2_ > Ⓢ*A*_5_ > Ⓢ*A*_1_

**Table 11:** Ranking of alternatives using IFDWG and TFDWG operators.

IFDWG operator	Ⓢ*A*_1_ > Ⓢ*A*_2_ > Ⓢ*A*_5_ > Ⓢ*A*_3_ > Ⓢ*A*_4_
TFDWG operator	Ⓢ*A*_3_ > Ⓢ*A*_4_ > Ⓢ*A*_2_ > Ⓢ*A*_5_ > Ⓢ*A*_1_

**Table 12:** Bipolar fuzzy (BF) decision matrix.

BF matrix values
$M^{\prime \prime }=\left[\begin{array}{cccc} \left(0.7,-0.3\right) & \left(0.2,-0.8\right) & \left(0.2,-0.3\right) & \left(0.8,-0.2\right)\\ \left(0.6,-0.4\right) & \left(0.3,-0.5\right) & \left(0.5,-0.4\right) & \left(0.4,-0.6\right)\\ \left(0.4,-0.2\right) & \left(0.4,-0.1\right) & \left(0.3,-0.5\right) & \left(0.5,-0.4\right)\\ \left(0.2,-0.6\right) & \left(0.3,-0.7\right) & \left(0.4,-0.2\right) & \left(0.5,-0.3\right)\\ \left(0.7,-0.3\right) & \left(0.5,-0.4\right) & \left(0.5,-0.4\right) & \left(0.4,-0.4\right) \end{array}\right]$

**Table 13:** Aggregated BFNs by using BFDWA and BFDWG operators.

Alternatives	BFDWA operator	BFDWG operator
*A*_1_	(0.0013, −0.9871)	(0.9875, −0.0004)
*A*_2_	(0.9959, −0.0004)	(0.0001, −0.9936)
*A*_3_	(0.0010, −0.9964)	(0.9674, −0.0008)
*A*_4_	(0.9944, −0.0015)	(0.0037, −0.9814)
*A*_5_	(0.0004, −0.8852)	(0.9984, −0.0003)

**Table 14:** Score values by using BFDWA and BFDWG operators.

Alternatives	BFDWA operator	BFDWG operator
*A*_1_	0.0071	0.9974
*A*_2_	0.0023	0.9964
*A*_3_	0.0576	0.9935
*A*_4_	0.0032	0.9833
*A*_5_	0.0111	0.9990

**Table 15:** Ranking of alternatives in BFDWA/BFDWG operators.

BFDWA operator	Ⓢ*A*_3_ > Ⓢ*A*_5_ > Ⓢ*A*_1_ > Ⓢ*A*_4_ > Ⓢ*A*_2_
BFDWG operator	Ⓢ*A*_5_ > Ⓢ*A*_1_ > Ⓢ*A*_2_ > Ⓢ*A*_3_ > Ⓢ*A*_4_

**Table 16:** Ranking of proposed and BFDWA/BFDWG operators.

BFDWA operator	Ⓢ*A*_3_ > Ⓢ*A*_5_ > Ⓢ*A*_1_ > Ⓢ*A*_4_ > Ⓢ*A*_2_
BFDWG operator	Ⓢ*A*_5_ > Ⓢ*A*_1_ > Ⓢ*A*_2_ > Ⓢ*A*_3_ > Ⓢ*A*_4_
TFDWA operator (proposed)	Ⓢ*A*_3_ > Ⓢ*A*_4_ > Ⓢ*A*_2_ > Ⓢ*A*_6_ > Ⓢ*A*_1_
TFDWG operator (proposed)	Ⓢ*A*_3_ > Ⓢ*A*_4_ > Ⓢ*A*_2_ > Ⓢ*A*_5_ > Ⓢ*A*_1_

**Table 17:** Comparison of proposed and existing methods.

Methods	Describe fuzzy information easier	More flexible by a parameter
Dombi [30]	Yes	No
Xu and Yager [5]	Yes	No
Proposed operator	Yes	Yes

## Data Availability

The data used in the manuscript are hypothetical and can be used by anyone by just citing this article.
